# An Improved New Caledonian Crow Learning Algorithm for Global Function Optimization

**DOI:** 10.1155/2022/9248771

**Published:** 2022-10-10

**Authors:** Yanjiao Wang, Jiaxu Song, Ziming Teng

**Affiliations:** ^1^Department of Electrical Engineering, Northeast Electric Power University, Jilin 132012, China; ^2^Department of Communication Engineering, Jilin University, Jilin 130012, China

## Abstract

The New Caledonian crow learning algorithm (NCCLA) is a novel metaheuristic algorithm inspired by the learning behavior of New Caledonian crows learning to make tools to obtain food. However, it suffers from the problems of easily falling into local optima and insufficient convergence accuracy and convergence precision. To further improve the convergence performance of NCCLA, an improved New Caledonian crow learning algorithm (INCCLA) is proposed in this paper. By determining the parent individuals based on the cosine similarity, the juveniles are guided to search toward different ranges to maintain the population diversity; a novel hybrid mechanism of complete and incomplete learning is proposed to balance the exploration and exploitation capabilities of the algorithm; the update strategy of juveniles and parent individuals is improved to enhance the convergence speed and precision of the algorithm. The test results of the CEC2013 and CEC2020 test suites show that, compared with the original NCCLA algorithm and four of the best metaheuristics to date, INCCLA has significant advantages in terms of convergence speed, convergence precision, and stability.

## 1. Introduction

A large number of optimization problems exist in real life, engineering design, computer technology and other fields, such as minimum cost, optimal parameters, minimum time, pipeline route design, welded beam design, etc. In order to obtain higher economic efficiency and social value, scholars strive to obtain the optimal solution to optimization problems, thus making the research of optimization methods widely concerned.

Optimization methods usually include traditional optimization methods such as the fastest descent method and metaheuristic methods. Among them, traditional optimization methods usually require the optimization problem to be derivable, and the convergence speed and convergence precision are difficult to meet the practical needs when the optimization problem has multiple extrema. And the metaheuristic algorithms proposed by simulating biological habits in nature, etc., have good exploration and exploitation performance through information exchange among individuals in the population. Compared with traditional optimization algorithms, metaheuristic algorithms are better in convergence speed, convergence precision, robustness, and stability, with no strict requirements on the form of optimization problems. This makes the metaheuristic algorithm the most effective and widely used optimization method. Researchers have focused on two main aspects of metaheuristics to obtain the best optimization results: improving existing metaheuristics and proposing new ones.

Various metaheuristic algorithms have been proposed, and the more representative methods are as follows: the artificial bee colony algorithm (ABC) was proposed to simulate the behavior of bee colonies to find the optimal nectar source according to different internal divisions of labor [1]; the crow search algorithm (CSA) was proposed to simulate the behavior of crows to hide and search for food [2]; particle swarm optimization (PSO) algorithm was proposed to simulate the foraging behavior of a flock of birds [3]; the firefly algorithm (FA) was proposed to simulate the behavior of fireflies to attract each other [4]; the Marine Predator Algorithm (MPA) was proposed to simulate the behavior of biological interactions between marine predators and prey [5]; the Manta Ray Foraging Optimization Algorithm (MRFO) was proposed to simulate three unique foraging modes of manta rays: chain foraging, cyclone foraging, and somersault foraging [6]; the dolphin swarm optimization algorithm (DSA) was proposed to simulate the habits of dolphins such as echolocation and information exchange [7]; and the gray wolf optimization algorithm (GWO) was proposed to simulate the hunting behavior of gray wolves [8] and so on. Some of the algorithms mentioned above have been applied to many research articles, such as applying particle swarm optimization to solve the UCP problem with deterministic and stochastic load demands [9], the ocean predator algorithm to solve the optimal reactive power dispatch (ORPD) problem [10], and the manta ray foraging optimization algorithm to solve the economic load dispatch and advance dispatches problems of microgrids [11].

Researchers have done a lot of work on the improvement of existing metaheuristic algorithms, and the more representative research results are given below. Many improvement methods for particle swarm algorithms have been proposed in recent years, and the representative results are as follows: In 2016, Samma et al. proposed the RLMPSO algorithm [12], where each particle performs five operations under the control of the RL algorithm to improve the search performance of the particle swarm algorithm. In 2018, Zhang et al. proposed the DLPSO algorithm [13] to address the shortcomings of the PSO algorithm in multimodal indivisible problems that tend to fall into local optima, which extracts good vectors from the vectors distributed in the search space to form a new vector with a greater possibility of jumping out of local optima. In 2021, Lu et al. proposed the EMCPSO algorithm [14], which takes advantage of the technology of multiple populations in order to overcome the problem of premature convergence of PSO, which divides the population into four identical subpopulations, and the optimal individual in each subpopulation is used to represent the evolutionary state of that subpopulation, and by sharing information among the four populations, the evolutionarily stagnant subpopulations search for the optimal solution again, while introducing an exclusion mechanism to prevent premature convergence of particles further. In 2022, Wang et al. proposed the RLLPSO algorithm for large-scale optimization problems [15], which constructs a level-based population structure to improve population diversity, a reinforcement learning strategy as well as a level competition strategy to improve the search efficiency of the algorithm in order to overcome the complexity of large-scale optimization problems.

Many improvement methods have been proposed for the artificial bee colony algorithm, and the representative results are as follows: In 2018, Cui et al. proposed the DPABC algorithm [16], which uses a dual population framework to divide the population into a convergence population and a diversity population, responsible for developing promising regions as well as maintaining population diversity, respectively, to improve the overall performance of the algorithm. In 2019, Awadallah et al. improved the onlooker bee stage [17], combining four selection methods, including global optimum, tournament, linear ranking, and exponential ranking, to guide the search process of the onlooker bee in order to determine the impact of the selection scheme on the onlooker bee stage. In 2021, Zhou et al. proposed the ABC-MNT algorithm [18], which applies three different neighborhoods to different individuals, helping the algorithm to achieve a better balance between exploration and exploitation, in addition to employing a global neighborhood search strategy and opposition-based learning that preserves the search experience of the scout bee phase. In 2022, Ye et al. proposed the RNSABC algorithm [19], which uses a random neighborhood structure so that each solution has a random neighborhood, in addition to a depth-first search method to enhance the search capability of the following bee to improve the algorithm's ability to search for the optimal solution.

Representative results of the improvement of other mainstream metaheuristic algorithms are as follows: In 2017, Wang et al. proposed a firefly algorithm with neighborhood attractiveness (NaFA) [20], where each firefly selects attractive individuals from a predefined region instead of the whole population, and the proposed strategy can effectively improve the solution accuracy and reduce the time complexity. In 2018, Sun et al. proposed an improved whale optimization algorithm (MWOA) for solving large-scale optimization problems [21], which uses a nonlinear dynamic strategy based on the cosine function to update the control parameters, balances the exploration and exploitation capabilities of the algorithm, uses a Levy flight strategy to make the algorithm jump out of the local optimum, and uses quadratic interpolation for the optimal individuals of the population to enhance the local exploitation capabilities of the algorithm. In 2019, Zamani et al. proposed a conscious neighborhood-based crow search algorithm (CCSA) [22], which introduces three search strategies, neighborhood-based local search strategy, non-neighborhood global search strategy, and roaming-based search strategy, to enhance the balance between local and global search. In 2020, Gupta et al. proposed a memory-based gray wolf optimization algorithm (mGWO) [23], which modified crossover and greedy selection based on the historical optimum of individuals, enhancing the algorithm's ability to perform the global search, local exploitation, and the balance between the two. In 2022, Long et al. proposed a velocity-based butterfly optimization algorithm (VBOA) [24], which introduced velocity and memory to guide individuals in the local search phase and introduced a refraction-based learning strategy, effectively enhancing the diversity of populations and the exploration ability of the algorithm.

Many excellent metaheuristic algorithms have been proposed in recent years. In 2018, Wang proposed the moth search algorithm (MSA) [25] inspired by the phototropism of moths and Levy flight, which treats moths as individuals. Moths with smaller distances from the optimal individual perform Levy flight, while moths with more considerable distances approach the optimal individual in a straight line. The above two stages optimize the algorithm. In 2019, Heidari et al. proposed the Harris Hawk optimization algorithm (HHO) [26] based on the inspiration of the collaborative group behavior of Harris hawks during predation, which uses Harris hawks as individuals, and the search process includes three stages: exploration, exploration to exploitation conversion, and exploitation, and the algorithm is characterized by few control parameters and excellent global search capability. In 2020, Li et al. proposed the slime mold algorithm (SMA) [27], inspired by the behavioral and morphological changes in *Physarum polycephalum* during foraging, which creates three different forms to optimize the problem by using weights to simulate the positive and negative feedback generated by slime molds during foraging. In the same year, Al-Sorori and Mohsen proposed the New Caledonian crow learning algorithm (NCCLA) [28] based on the behavior of New Caledonian crows to obtain food by learning to make tools. The advantage of this algorithm is its stochastic nature, which guarantees that the algorithm does not get trapped at the local optimum. In the same year, Mohamed et al. proposed a gaining-sharing knowledge-based algorithm (GSK) [29] inspired by the process of acquiring and sharing knowledge in the human life cycle, which treats people as individuals and improves their knowledge by using junior gaining and sharing phase and senior gaining and sharing phase, i.e., solving optimization problems on continuous space. In 2021, Tu et al. proposed the colony predation algorithm (CPA) [30], inspired by the supportive behavior of herd animals and the behavior of selective hunting, which is based on the coexistence of social animals and focuses on optimizing the problem through five stages: communicating and collaborating, dispersing food, surrounding food, supporting the closest individual, and finding food. In 2022, Hashim et al. proposed the snake optimizer (SO) [31], based on the behavior of snakes to forage or breed under different temperature and food availability conditions, in which individuals explore and exploit the conditions of temperature as well as food.

The various metaheuristic algorithms mentioned above provide new ideas for solving optimization problems and further advance the development of optimization techniques. Compared with the more classical PSO and DE, they have significantly improved in terms of convergence speed and convergence precision. However, unfortunately, for the highly nonlinear and complex optimization problems that emerge one after another in practical engineering, the convergence speed and convergence precision of the existing metaheuristic algorithms are obviously insufficient and even fall into local optimum, making it difficult to obtain highly satisfactory economic and social values. Therefore, improving the optimization performance of each new metaheuristic algorithm has been one of the main research contents in the field of evolution.

In this context, given the literature [28] and a large number of experimental studies, the NCCLA algorithm is a very excellent metaheuristic algorithm because of its simple operation and significantly better convergence capability than optimization algorithms such as GWO, CSA, and WOA, and is highly promising in fields such as engineering optimization. In this paper, we only study NCCLA. In order to further improve the problems of insufficient convergence precision and convergence speed and easy falling into local optimum when NCCLA deals with very complex optimization problems, we propose an improved New Caledonian Crow Learning Algorithm (INCCLA) in this paper.

The main innovations and contributions of INCCLA are as follows: (1) A cosine similarity-based parent individual selection approach is proposed. The globally optimal individual and another excellent individual with a significant difference in similarity are selected as the parent, and the juvenile crow individuals are guided to search toward different ranges to maintain the population diversity while maintaining the convergence speed of the algorithm. (2) Improving the learning phase of juvenile crows. A new hybrid learning mechanism of complete learning and incomplete learning is set up, in which the individual juvenile crows in the complete learning stage can select learning objects according to their own conditions, which effectively improves the convergence speed of the algorithm while maintaining the population diversity to a certain extent; while the juvenile crows in the incomplete learning stage learn the behavioral attributes of different individuals in order to maintain the population diversity of the algorithm. (3) Improving the reinforcement phase. For the juvenile reinforcement stage, a weighting factor is introduced to enable the algorithm to have a strong exploration ability in the early evolutionary stage and a strong exploitation ability in the late evolutionary stage, and at the same time, a small range of random perturbations is added to increase the possibility of convergence of the algorithm to the global optimum; for the parents' reinforcement stage, the update methods of the two parents' individuals are improved further to respectively balance the exploration and exploitation ability of the algorithm. The results of testing on the CEC2013 and CEC2020 test suites show that the INCCLA proposed in this paper has significant advantages in terms of convergence speed, convergence precision, and stability compared with four other more representative optimization algorithms.

The rest of the paper is organized as follows: Section 2 describes the working principle and flow of the NCCLA algorithm.  Section 3 analyzes the defects of the original NCCLA algorithm and further proposes an improved INCCLA algorithm.  Section 4 shows the simulation results and analysis of the INCCLA algorithm with the original NCCLA algorithm and other more mainstream improved algorithms on the CEC2013 and CEC2020 test function suites.  Section 5 concludes the proposed algorithm in this paper.

## 2. New Caledonian Crow Learning Algorithm

In nature, New Caledonian crows are divided into the juvenile and the parent crows, which enhance their tool-design skills through learning and their own experience and knowledge, respectively, to obtain food from the pandanus tree. Inspired by the above behavior, Wedad and Abdulqader proposed the New Caledonian crow learning algorithm (NCCLA). In NCCLA, individuals represent the manufacturing behavior of New Caledonian crows and fitness values represent the behavioral advantage of each crow. The algorithm has three main phases: initialization, learning phase, and reinforcement phase. The pseudo-code of NCCLA is shown in Algorithm 1, and the key steps are briefly described as follows.

### 2.1. Population Initialization

Suppose the number of individuals in population *X* is *N*. Each individual *X*_*i*_ (*i* = 1, 2,…, *N*) represents the behavior of a crow, which can be expressed as *X*_*i*_ = [*X*_*i,*1_, *X*_*i,*2_, *X*_*i,*3_,…, *X*_*i,D*_], where D is the dimension of the optimization problem, and *X*_*i,j*_ denotes the *j*-th behavioral attribute of the *i*-th crow. At the beginning of the algorithm, the initial behavior of each crow is generated randomly according to Equation.

(1) $$\begin{array}{c} X_{i,j}\left(0\right)=X_{L}+U\left(0,1\right)\times \left(X_{U}-X_{L}\right), \end{array}$$

where *X*_*U*_ and *X*_*L*_ correspond to the upper and lower bounds of the *j*-th dimensional search space in the optimization problem, respectively, and *U* (0,1) is a uniformly distributed random number in the range [0,1].

### 2.2. Learning Phase

In NCCLA, only juveniles enter the learning phase, and each behavioral attribute *X*_*i,j*_ of juveniles will be socially or asocially learned according to the probability SL_prob_ or 1-SL_prob_, respectively. SL_prob_ is recommended to be set to 0.95, but can be set to other values.

#### 2.2.1. Social Learning

After the *j*-th behavioral attribute of juvenile crow *i*, *X*_*i,j*_, is determined to require social learning according to the probability SL_prob_, it is then decided to perform vertical learning or horizontal learning according to the predetermined probability VSL_prob_ or 1 − VSL_prob_. The details are shown in Equation.

(2) $$\begin{array}{c} X_{i,j}\left(t\right)=\left\{\begin{array}{c} X_{k_{1},j}\left(t-1\right),\;\text{if rand}\leq VSL_{\text{prob}},\\ X_{k_{2},j}\left(t-1\right),\;\text{else}, \end{array}\right. \end{array}$$

where *X*_*i*,*j*_(*t*) is the *j*-th new behavioral attribute acquired by juvenile crow *i* after social learning in iteration *t*, VSL_prob_ is recommended to be set to 0.99, and can also be set to other values.

In (2), when rand ≤ VSL_prob_, the juvenile crow *X*_*i*_ performs vertical learning to its parent, i.e., it copies the corresponding behavioral attributes of its parent *X*_*p*1_ or *X*_*p*2_ with probability *P*1_prob_, obviously *k*_1_ = 1 or 2; Otherwise, the juvenile crow *X*_*i*_ performs horizontal learning, i.e., it randomly selects a sibling *k*_2_ that is more experienced and copies its corresponding behavioral attributes, and the expression formula for *k*_2_ is shown in equation (3). It should be noted that for the juvenile crow with the best fitness value, only vertical learning is performed, not horizontal learning.

(3) $$\begin{array}{c} k_{2}=3+\left[\text{rand}\times \left(i-3\right)\right], \end{array}$$

where rand is a random number uniformly distributed in the range [0, 1], [*·*] means rounding is performed.

#### 2.2.2. Asocial Learning

When a crow *X*_*i*_ performs asocial learning, its behavioral attributes are randomly updated using (1) according to the probability TaE_prob_, or retained the previous behavioral attributes according to 1 − TaE_prob_. This is shown in Equation .

(4) $$\begin{array}{c} X_{i,j}\left(t\right)=\left\{\begin{array}{c} X_{L}+U\left(0,1\right)\times \left(X_{U}-X_{L}\right),\;\text{rand}\leq TaE_{\text{prob}},\\ X_{i,j}\left(t-1\right),\;else, \end{array}\right. \end{array}$$

where TaE_prob_ is recommended to be set to 0.99, but can also be set to other values.

### 2.3. Reinforcement Phase

After completion of the learning phase, certain attributes of the learned juvenile crow behavior and parent behavior are reinforced according to the reinforcement probability RP_prob_. RP_prob_ is recommended to be set to 0.99, and can be set to other values.

#### 2.3.1. Juvenile Reinforcement

Each behavioral attribute of juvenile crows was reinforced according to Equation.

(5) $$\begin{array}{c} X_{i,j}\left(t\right)=X_{i,j}\left(t\right)\pm RW, \end{array}$$

where *RW* is shown in Equation.

(6) $$\begin{array}{c} RW=\left\{\begin{array}{c} \beta -\alpha ,\;i<N,\\ r1\times \left(\left(r2\times \beta \right)-\alpha \right),\;\text{otherwise}, \end{array}\right. \end{array}$$

where *r*1 and *r*2 are random numbers between 0 and 1, *α* represents the difference between their behavioral attributes before and after learning, as shown in (7), and *β* represents the social learning effect developed over time, as shown in Equation (8).

(7) $$\begin{array}{c} \alpha =\left|X_{i,j}\left(t\right)-X_{i,j}\left(t-1\right)\right|, \end{array}$$

(8) $$\begin{array}{c} \beta =X_{i,j}\left(t-1\right)\times e^{-lf\times r\times t\times \text{mean}\left(j\right)}, \end{array}$$

where *t* represents the number of current iterations, *X*_*i,j*_ (*t* − 1) is the *j*-th behavioral attribute of crow *i* before the current generation of learning, *r* is a normally distributed random number in the range [0,1], mean (*j*) is the average of the *j*-th behavioral attribute of all individuals in the population, and lf is a learning factor, as shown in Equation .

(9) $$\begin{array}{c} lf=lf_{\min}+\left(\frac{\left(lf_{\max}-lf_{\min}\right)}{\max\_t}\right)\times t, \end{array}$$

where max_*t* represents the maximum number of iterations, lf_max_ and lf_min_ represent the maximum and minimum values of the learning factor, respectively, and are recommended to be set to 0.02 and 0.0005, respectively, or can be set by oneself.

#### 2.3.2. Parents Reinforcement

The parents *X*_*p*1_ and *X*_*p*2_ update certain attributes according to the reinforcement probability RP_prob_. When rand ≤ RP_prob_, the *j*-th dimensional behavioral attribute of crow *i* is reinforced, as shown in (10); otherwise, it retains the original behavioral attribute.

(10) $$\begin{array}{c} X_{i,j}\left(t\right)=\left\{\begin{array}{c} X_{i,j}\left(t-1\right)-\left(X_{1,j}\left(t-1\right)+e^{r1\times \left(\text{mean}\left(j\right)-X_{i,j}\left(t-1\right)\right)}\right),\;\;\;\;i=p1,\\ X_{i,j}\left(t-1\right)-\left(r2\times \left(X_{1,j}\left(t-1\right)-e^{r1\times \left(\text{mean}\left(j\right)-X_{i,j}\left(t-1\right)\right)}\right)\right),\;i=p2, \end{array}\right. \end{array}$$

where *r*1 is a normally distributed random number, *r*2 is a uniformly distributed random number in the range [0, 1], and mean (*j*) is the mean of the *j*-th behavioral attribute of all individuals in the current population.

## 3. Proposed Algorithm

To further improve the convergence performance of NCCLA, this section proposes an improved New Caledonian Crow Learning Algorithm (INCCLA), whose pseudo-code is shown in Algorithm 2.

### 3.1. Determination of Parent Individuals Based on Cosine Similarity

In NCCLA, VSL_prob_ and P1_prob_ are set to 0.99 and 0.95, respectively, meaning that each juvenile crow will perform vertical learning with a probability of 0.99 × 0.95 toward the parent individual during the learning phase. The parent individuals are always the two individuals with the best fitness in the population. As evolution proceeds, the two-parent individuals will rapidly approach each other, showing a high degree of similarity, which will lead most of the juvenile crows to approach them through vertical learning rapidly, and can only search around the parent individuals, lacking exploration of other ranges. Although rapid convergence can be achieved in the early stage of evolution, the loss of population diversity is apparent, and the algorithm is straightforward to fall into the local optimum.

In order to solve the above problem, the following cosine similarity-based parent individual selection method is proposed in this section. First, the best individual in the population is determined as the parent individual *X*_*p*1_; then, the cosine similarity of the remaining individuals in the population to *X*_*p*1_ is calculated according to (11), and they are arranged in order from smallest to largest and evenly divided into two groups; finally, the individual with the best fitness value is selected as the parent individual *X*_*p*2_ from the other group different from the group in which *X*_*p*1_ is located. It is important to note that the parent individuals are selected for every *P* generation above. Generally, *P* = 50 is sufficient to achieve good results, but it can also be set according to the optimization problem.

(11) $$\begin{array}{c} sim_{i,p1}\left(t-1\right)=\frac{\sum_{j=1}^{D}X_{p1,j}\left(t-1\right)\times X_{i,j}\left(t-1\right)}{\sqrt{\sum_{j=1}^{D}{\left(X_{p1,j}\left(t-1\right)\right)}^{2}}\times \sqrt{\sum_{j=1}^{D}{\left(X_{i,j}\left(t-1\right)\right)}^{2}}},\;i=1,2,...,N, \end{array}$$

where *X*_*p*1*,j*_ (*t* − 1) denotes the *j*-th dimension of the globally optimal individual *X*_*p*1_ (*t* − 1) determined by relying on the previous iteration of the population, and sim_*i,p*1_ (*t* − 1) denotes the cosine similarity of the *i*-th individual *X*_*i*_ (*t* − 1) without any evolutionary operation to *X*_*p*1_ (*t* − 1) in the current generation.

To further illustrate the above method of determining parent individuals based on cosine similarity, taking the optimized 2-dimensional Rotated High Conditioned Elliptic function as an example, the specific determination process is given in Figure 1. It can be seen that, according to the original parent individual determination method, *X*_1_ and *X*_2_, which are close to each other, will be selected as parent individuals, while according to the proposed method in this section, *X*_1_ and *X*_4_, which are farther apart, will be selected as parent individuals. The fitness value of *X*_4_ is not much worse than *X*_2_.

In summary, compared with the original approach of selecting two more similar optimal individuals as parents, this section retains the optimal individual of the population as a parent individual, which does not affect the convergence speed too much. In contrast, the other parent individual is selected to be less similar to the optimal individual of the population but with better fitness value. This way can guide juveniles in their search across a range and ensure that they learn from more experienced individuals, maintaining good population diversity while not reducing the convergence speed too much.

### 3.2. Improving Juvenile Crow Learning Phase

As seen in Algorithm 1, the learning phase generates its own learning objects for juvenile crows intending to provide excellent evolutionary directions for the reinforcement phase. In-depth analysis can be found that the various behavioral attributes of the learning objects generated in the learning phase are not almost wholly derived from the same individual. Although the population diversity can be better maintained, it is difficult to ensure the superiority of the learning objects composed of them due to the complete separation of each behavioral attribute. Therefore, it is difficult to guarantee the convergence speed of the reinforcement phase. The excellent individuals themselves are already better integrated with each behavioral attribute, which has a vital role in the rapid convergence of the algorithm but is not conducive to the maintenance of population diversity. Given this, this section proposes a novel juvenile learning approach as shown in Figure 2. *R* juveniles are randomly selected to perform complete learning, i.e., each behavioral attribute of the corresponding learning object originates from the same individual completely, which promotes fast convergence of the algorithm; while the remaining juveniles perform incomplete learning, i.e., each behavioral attribute of the learning object originates from different individuals, which ensures population diversity.

#### 3.2.1. Complete Learning

As mentioned above, the complete learning phase aims to enhance the convergence speed of the algorithm by copying all the behavioral attributes of a particular outstanding individual. In contrast to social learning, asocial learning focuses on maintaining population diversity; therefore, in the complete learning phase, asocial learning is eliminated, and only social learning is used.

Social learning in NCCLA includes vertical and horizontal learning, where vertical learning is learning from the two best parent individuals in the population, while horizontal learning is learning from other individuals who are better than oneself. Obviously, compared with vertical learning, horizontal learning is more capable of maintaining population diversity. In NCCLA, vertical or horizontal learning is chosen according to the fixed probability VSL_prob_. If VSL_prob_ is high, the population will quickly approach the parent individuals, accelerating the algorithm's convergence. However, the rapid loss of population diversity can easily cause the algorithm to fall into local optimum. If VSL_prob_ is low, each individual may have different learning objects, and introducing multiple learning objects makes the evolutionary direction of each individual more diffuse, which is not conducive to the rapid convergence of the population. The NCCLA recommends that VSL_prob_ be set to 0.95, allowing all juveniles to primarily use vertical learning as their social learning method. In vertical learning, individuals need to choose to learn from the best parent *X*_*p*1_ or the second-best parent *X*_*p*2_ according to the fixed probability SL_prob_. If SL_prob_ is large or small, all juvenile crows will search around a parent almost exclusively, which is not conducive to the maintenance of population diversity and increases the possibility of the algorithm falling into local optimum; If SL_prob_ is set to about 0.5, it will learn from the parent individuals with equal chances, which is similar to random selection and has certain blindness, slowing down the convergence of the algorithm to some extent. In short, the selection methods of vertical learning or social learning by fixed probability and the selection of a certain parent individual for learning by fixed probability in vertical learning are not very reasonable.

Given this, to effectively improve the convergence speed of the algorithm and not destroy the population diversity too much, we propose the complete social learning method as shown in Equation.

(12) $$\begin{array}{c} X_{i}\left(t\right)=\left\{\begin{array}{c} X_{k_{1}}\left(t-1\right),\;if\;F_{i}\left(t-1\right)\leq {\bar{F}}_{i}\left(t-1\right)\&sim_{i,p1}\left(t-1\right)\geq \bar{sim_{i,p1}\left(t-1\right)}\\ X_{k_{2}}\left(t-1\right),\;else \end{array}\right., \end{array}$$

where *F*_*i*_ (*t* − 1) denotes the fitness value of juvenile *X*_*i*_, $\bar{F_{i}}\left(t-1\right)$ denotes the mean of the fitness values of all individuals in the population, sim_*i,p*1_ (*t* − 1) denotes the cosine similarity of juvenile *X*_*i*_ to the best individual *X*_*p*1_ in the population. $\bar{sim_{i,p1}\left(t-1\right)}$ denotes the mean of the cosine similarity of all individuals in the population to *X*_*p*1_. When both $F_{i}\left(t-1\right)\leq \bar{F_{i}\left(t-1\right)}$ and $sim_{i,p1}\left(t-1\right)\geq \bar{sim_{i,p1}\left(t-1\right)}$ are satisfied, the juvenile *X*_*i*_ performs vertical learning from the parent *X*_*p*1_ or *X*_*p*2_ according to (13); otherwise, the juvenile *X*_*i*_ will perform horizontal learning in the original way of NCCLA, i.e., it randomly selects a juvenile with a better adaptation value than itself as the learning object.

(13) $$\begin{array}{c} X_{i}\left(t-1\right)=\left\{\begin{array}{c} X_{p1}\left(t-1\right),\;if\;\frac{e^{-sim_{i,p1}\left(t-1\right)}}{1+e^{-5\times NF_{p1}}}\geq \frac{e^{-sim_{i,p2}\left(t-1\right)}}{1+e^{-5\times NF_{p2}}},\\ X_{p2}\left(t-1\right),\;else, \end{array}\right. \end{array}$$

where sim_*i,p*1_ and sim_*i,p*2_ denote the cosine similarity of juvenile *X*_*i*_ to the parent individuals *X*_*p*1_ and *X*_*p*2_, respectively, and NF_*i*_ denotes the normalization ability of juvenile *X*_*i*_ as shown in equation (14). The better the individual fitness value, the stronger its normalization ability.

(14) $$\begin{array}{c} NF_{i}=\left\{\begin{array}{c} \left|\frac{\max\left(F\right)-F_{i}}{\sum_{i=1}^{N}F_{i}}\right|,\;if\;\sum_{i=1}^{N}F_{i}\neq 0,\\ \frac{1}{N},\;else. \end{array}\right. \end{array}$$

In summary, this section proposes the complete social learning approach with the following advantages. First, compared with the original fixed-probability selection of vertical or horizontal learning, the new selection approach proposed in this section, as shown in (12), can rely on individuals' conditions to adaptively select the learning mode. Only juvenile individuals with convergence potential, i.e., those who are more similar to the optimal individuals and have better fitness values, will perform vertical learning. In contrast, the rest of the individuals will perform horizontal learning. Obviously, this approach makes a small number of dominant individuals, who are not far from the optimal parent and are more excellent, focus on mining in the region with more convergence prospects and then quickly determine the more excellent evolutionary direction, driving the rapid convergence of the rest individuals. In turn, most of the remaining individuals learn from other better juvenile crows, which can develop other search areas, facilitating the maintenance of population diversity and reducing the risk of the algorithm falling into a local optimum. Second, the new vertical learning approach as shown in (13)proposed in this section, which relies on a comprehensive judgment of individual fitness values and the degree of similarity with individuals of the two parents, selects individuals learning from the parent with less similarity and excellent performance, and enables the juvenile crows to explore different promising areas as much as possible, which can better maintain the population diversity while ensuring the convergence speed. In short, the complete learning approach proposed in this section selects the learning mode and learning objects in a targeted way according to the juvenile crows' conditions, which effectively improves the convergence speed of the algorithm and maintains the population diversity to a certain extent. In addition, the above process no longer uses the parameters VSL_prob_ and SL_prob_, which avoids the trouble of parameter debugging.

#### 3.2.2. Incomplete Learning

As mentioned above, the incomplete learning phase will generate new learning objects by copying and absorbing the behavioral attributes of different individuals. To further ensure that the algorithm maintains population diversity and avoids falling into local optimum while improving the convergence speed, this section improves the asocial learning behavior and social learning behavior in the original NCCLA separately and proposes a new incomplete learning approach. The details are as follows.

(1) Improvement of social learning behavior
This section improves the conditions of vertical and horizontal learning in the social learning approach in NCCLA, as well as the horizontal learning approach, and proposes a new incomplete social learning approach as follows. First, the adaptive selection factor *δ*_*i*_(*t*) is calculated for the *i*-th juvenile crow individual *X*_*i*_ as shown in (15); then, a random number rand between [0,1], and if rand ≤ *δ*_*i*_(*t*) is generated, vertical learning is performed, i.e., the behavioral attributes corresponding to the *j*-th dimension of the parent individual *X*_*p*1_ or *X*_*p*2_ as shown in equation (13) are copied, otherwise, horizontal learning is performed, i.e., the behavioral attributes of the *j*-th dimension of the individual shown in equation (16) are copied.
  (15) $$\begin{array}{c} \delta_{i}\left(t\right)=1-e^{-\left|F_{i}\left(t-1\right)-F_{gbest}\left(t-1\right)\right|}, \end{array}$$
where *F*_*gbest*_(*t* − 1) and *F*_*i*_(*t* − 1) represent the fitness values of the globally optimal individual and the juvenile *Xi* before the current generation's juvenile crow learning operation, respectively.
  (16) $$\begin{array}{c} X_{i,j}\left(t\right)=\left\{\begin{array}{c} X_{s,j}\left(t-1\right),\;if\text{ rand}\leq 0.5,\\ \frac{X_{p1,j}\left(t-1\right)+X_{r1,j}\left(t-1\right)+X_{r2,j}\left(t-1\right)}{3},\;else, \end{array}\right. \end{array}$$
where *X*_*p*1_ is the optimal parent individual, *X*_*r*1_ is a randomly selected individual with a better fitness value than the juvenile crow *X*_*i*_, *X*_*r*2_ is a randomly selected individual in the population, and *X*_*s*_ is the individual selected among all juvenile crow individuals using roulette selection according to the probability corresponding to equation (17).
  (17) $$\begin{array}{c} P_{k}\left(t\right)=\frac{e^{-sim_{i,k}\left(t-1\right)}}{1+e^{-5\times NF_{k}}}, \end{array}$$
where sim_*i,k*_ denotes the cosine similarity between the juvenile crow *X*_*i*_ and the juvenile crow *X*_*k*_ before learning was performed, and NF_*k*_ denotes the normalization ability of the juvenile crow *X*_*k*_.
(2) Improvement of asocial learning behavior
In NCCLA, the probability of asocial learning behavior occurring is only 1-VSL_prob_ × *P*1_prob_, which is only 1 − 0.99 × 0.95 by its proposed parameter setting. In essence, such a small probability of asocial learning behavior occurring is intended to provide new evolutionary genes and reduce the possibility of the algorithm falling into a local optimum. Obviously, there is no need to keep certain properties unchanged with a certain probability. For this reason, the asocial learning in the incomplete learning phase only randomly updates each behavioral attribute according to equation (1).
The analysis shows that the incomplete learning approach proposed in this section has the following advantages. First, each behavioral attribute of new juvenile individuals after incomplete learning may originate from different individuals, including parent individuals *X*_*p*1_ and *X*_*p*2_, any other individual in the population, and new genes generated by asocial learning, forming various combinations that can ensure excellent population diversity. Second, the incomplete learning phase mainly uses incomplete social learning and rarely uses asocial learning. Compared with the original social learning approach, the new social incomplete learning proposed in this section better adapts to the needs of the algorithm performance at different stages of the algorithm, as follows: at the early stage of evolution, the individuals in the population are more distributed, with better population diversity, and the difference between individuals and optimal individuals is large. According to the adaptive selection factor, most of the dimensions of the new individuals come from the parent individuals, and a few dimensions come from other juvenile individuals, which further promotes the rapid convergence of the population; while in the late evolutionary stage, all individuals gradually approach the globally optimal individuals, the population shows a certain aggregation, and the population diversity decreases, at this time, most of the dimensions of the new individuals are derived from other more experienced juvenile individuals, which maintains the population diversity without slowing down the convergence of the algorithm. Third, when individuals perform horizontal learning in a certain dimension, they can no longer learn and communicate only with other juveniles who are better than themselves but have the opportunity to exchange information with any individual in the population, which further enhances population diversity, and learning from individuals who are less similar to and better than themselves based on roulette selection does not reduce the convergence speed while maintaining population diversity. In summary, the incomplete learning approach proposed in this section can indeed achieve the goal of maintaining population diversity and maximizing convergence speed.

### 3.3. Improvement in Reinforcement Phase

#### 3.3.1. Improvements of Juvenile Crows Reinforcement Phase

In fact, the juvenile crow reinforcement phase in NCCLA is an offset search of *RW* near the learning objectives identified in the juvenile crow learning phase. The offset range *RW* is a combination of *α* and *β*, where *α* represents self-perception and *β* represents social perception, which aims to enhance the exchange of evolutionary information with other individuals and thus explore more search space. The experimental study shows that the unreasonable settings of *RW* and *β* make the quality of the reinforced individuals still have much room for improvement, for which they are improved separately.

(1) Improvement of *β* calculation method
An in-depth analysis of (8) reveals that *β* is actually a reference to the information of other individuals and scales the individual itself by exp (−lf × *r* × *t* × mean (*j*)) times. As the number of iterations *t* increases, if mean (*j*) < 0, exp (−lf × *r* × *t* × mean (*j*)) will be huge, even tending to infinity. The corresponding *β* and *RW* are also extremely large, making it extremely easy for the reinforced individuals to exceed the search range, resulting in ineffective reinforcement and making it difficult to provide new individuals with more excellence, leading to slow convergence of the algorithm or even failure to converge to the global optimum. Given this, a new calculation of the social perception factor *β* is proposed, as shown in equation (18).
  (18) $$\begin{array}{c} \beta =\left(X_{i,j}\left(t-1\right)-X_{k,j}\left(t-1\right)\right)\times w\left(t\right), \end{array}$$
where *k* is a randomly selected individual different from *X*_*i*_ in the unlearned juvenile crow population, i.e., *i* ≠ *k*, and *w*(*t*) is a weighting factor, as shown in equation.
  (19) $$\begin{array}{c} w\left(t\right)=w_{\max}-\frac{w_{\max}-w_{\min}}{1+e^{-0.1\times r\times lf}}, \end{array}$$
where *w*_max_ and *w*_min_ are denoted as the maximum and minimum values of the weighting factors, respectively, generally, when *w*_max_ and *w*_min_ are 2 and 0, better results can be obtained.
The change process of the weight factor with iteration is shown in Figure 3. At the early stage of evolution, the weight factor maintains a large value, which disguisedly increases the social learning phase in the reinforcement phase. The communication between individuals is more extensive, which makes individuals search extensively in different regions, further enhancing the global search ability of individuals and reducing the risk of the algorithm falling into the local optimum; as the evolution proceeds, the weight factor gradually decreases, especially at the late stage of evolution, the weight factor maintains a small value for a long time, which weakens the communication between individuals and other individuals, and enhances the local exploration ability of individuals in their neighborhood, which is more conducive to finding the global optimum.
(2) Improvement of RW calculation method
An in-depth analysis of *RW* calculation, as shown in (6), reveals that when *α* and *β* are zero simultaneously, the reinforcement phase is ineffective and fails to provide new individuals. In practical optimization, the possibility of this situation is not low. For example, in the late stage of algorithm evolution, almost all individuals in the population will gather around the optimal individual, and the vast majority of them have similar behavioral attributes, or even some behavioral attributes of some individuals are entirely identical when *α* and *β* are likely to be zero at the same time. Obviously, in order to enable individuals to perform a refined search around the obtained optimal value and thus converge to the globally optimal position, when both *α* and *β* are zero at the same time, a new stochastic reinforcement strategy is proposed to calculate *RW* as shown in equation (20). Here, it should be noted that when *α* and *β* are not zero simultaneously, *RW* is still calculated according to the original way shown in equation (6).
  (20) $$\begin{array}{c} RW=r\times \left(X_{s1,j}\left(t-1\right)-X_{s2,j}\left(t-1\right)\right), \end{array}$$
where *s*1 and *s*2 are two different individuals randomly selected in the unlearned juvenile crow population, i.e., *s*1 ≠ *s*2 ≠ *i*, and *r* is a random number uniformly distributed in the range [0, 1].

As seen in (20), when the individuals within the population are more similar, the above random reinforcement strategy makes the individuals perform a small random perturbation near themselves, increasing the possibility of convergence of the algorithm to the global optimum.

#### 3.3.2. Improvements of Parent Crows Reinforcement Phase

In NCCLA, the parent individuals in this iteration are the two relatively better individuals identified in the previous iteration of the population, which directly guide the evolution of the current generation of juveniles play an important role in the exploration and exploitation of the algorithm. As seen from the parent reinforcement phase in Section 2.3, the two-parent individuals each self-update in their independent reinforcement according to the probabilistic RP_prob_. Further simplification reveals that the parent individuals *X*_*p1*_ and *X*_*p2*_ perform the reinforcement operation according to Equations 21 and 22.

(21) $$\begin{array}{c} X_{p1,j}\left(t\right)=e^{r1\times \left(\text{mean}\left(j\right)-X_{p1,j}\left(t-1\right)\right)}, \end{array}$$

(22) $$\begin{array}{c} X_{p2,j}\left(t\right)=X_{2,j}\left(t-1\right)-r2\times X_{1,j}\left(t-1\right)+e^{r1\times \left(\text{mean}\left(j\right)-X_{p2,j}\left(t-1\right)\right)}. \end{array}$$

Both of these reinforcement methods include *e*^*r*1×(mean(*j*) − *X*_*p*i,*j*_(*t* − 1))^. From the properties of the *e* exponential function, we can find that the effect of *e*^*r*1×(mean(*j*) − *X*_*p*i,*j*_(*t* − 1))^ is to amplify the gap between mean (*j*) and the two-parent individuals, especially when mean(*j*) − *X*_*i*,*j*_(*t* − 1) > 0, the gap amplification is more pronounced. In general, early in evolution, individual distribution is extremely dispersed, and the gap between individuals is not small, which is easily exceeded by the search space of the optimization problem after exponential amplification, resulting in ineffective reinforcement and waste of computational resources. Moreover, in the late stage of evolution, although the gap between individuals is not large, the further amplification of the gap by *e*^*r*1×(*mean*(*j*) − *X*_*i*,*j*_(*t* − 1)) ^ will cause the parent individuals to produce a not small offset in this dimension, which is also very easy to deviate from the excellent evolutionary direction and will likewise cause ineffective reinforcement. Obviously, the reinforcement mentioned above of the two-parent individuals cannot effectively meet the needs of algorithm evolution. Given the different roles of the two-parent individuals in the algorithm, the reinforcement methods of these two-parent individuals are improved separately further to balance the exploration and exploitation capabilities of the algorithm.

(1) Novel reinforcement of parent individual *X*_*p*1_
The parent individual *X*_*p*1_ is the optimal individual determined by relying on the previous iteration of the population, which plays a vital role in guiding the algorithm's convergence. However, if its evolutionary direction points directly to the optimum local peak, it will increase the possibility of the algorithm falling into the local optimum. In view of the fact that the juvenile individuals of this generation have already achieved self-improvement based on the two more excellent parent individuals, carrying more excellent evolutionary information, which can provide more excellent reference information for the parent individuals to determine the evolutionary direction, a novel reinforcement was designed for the first parent individual *X*_*p*1_ as shown in Equation .
  (23) $$\begin{array}{c} X_{p1,j}\left(t\right)=\left\{\begin{array}{c} X_{p1,j}\left(t-1\right)+G_{1}\times \left(\text{mean}\left(j\right)-X_{p1,j}\left(t-1\right)\right),\;if\;X_{p1,j}\left(t-1\right)\neq X_{k,j}\left(t\right)\\ X_{p1,j}\left(t-1\right)+r1\times e^{\frac{-16t^{2}}{\max\_t^{2}}}\times \left(X_{p1,j}\left(t-1\right)-X_{k,j}\left(t\right)\right),\;else \end{array}\right., \end{array}$$
where *r*1 is a random number uniformly distributed in the range [−1.5, 1.5], *X*_*k,j*_ (*t*) is the *j*-th behavioral attribute of a randomly selected individual different from *X*_*p*1_ (*t* − 1) in the current population, and *G*_1_ is a number conforming to the Gaussian distribution *N*∼(*X*_*p*1_,_*j*_ (*t* − 1),1), as shown in Equation
  (24) $$\begin{array}{c} G_{1}=\frac{1}{\sqrt{2\pi }}\times e^{\frac{-{\left(\text{mean}\left(j\right)-X_{p1,j}\left(t-1\right)\right)}^{2}}{2}}. \end{array}$$
From the above novel reinforcement approach for the parent individual *X*_*p*1_, it can be seen that if for the *j*-th dimension of *X*_*p*1_ relying on the probability RP_prob_ determines that reinforcement is needed, an individual *X*_*k*_ (*t*) needs to be randomly selected from the current population. By comparing whether *X*_*k,j*_ (*t*) is equal to *X*_*p*1,*j*_ (*t* − 1), it is determined that learning toward the mean (*j*) or *X*_*k,j*_ (*t*) is performed. At the early stage of evolution, *X*_*k,j*_ (*t*) is almost not equal to *X*_*p*1,*j*_ (*t* − 1). The *j*-th dimension of *X*_*p*1_ is reinforced by learning from *X*_*k,j*_ (*t*). Since the individuals in the current population already carry more excellent evolutionary information, the optimal evolutionary direction can be determined as soon as possible with reference to their evolutionary direction. As evolution proceeds, the range *r*1 × *e*^−16*t*^2^/max_*t*^2^^ of *X*_*p*1_ tries to explore a more optimal region gradually decreases, and gradually locks in a smaller range near the optimal individual to exploit a more optimal individual. This is in accordance with the process and law of evolutionary algorithms that gradually approach the region where the global optimal solution is located, avoiding the phenomenon of missing the optimal solution due to too large a search range. In addition, because the individuals of *X*_*p*1_ reinforcement learning are not the same on each behavioral attribute, it further enriches the range of dominant regions that can be explored by *X*_*p*1_, increasing the possibility of the algorithm locking the actual optimal region and reducing the risk of the algorithm falling into a local optimum due to a single evolutionary direction. Moreover, as evolution proceeds, individuals are more similar by the late stage of evolution, and the *j*-th dimension of *X*_*p*1_ will be reinforced with a high probability by learning from mean (*j*). Compared with *X*_*k,j*_ (*t*), the *j*-th dimension of *X*_*p*1_ is more likely to be different from mean (*j*), and the difference between mean (*j*) and the *j*-th dimension of *X*_*p*1_ is smaller, making the optimal individual *X*_*p*1_ able to perform a more refined search within the current range, making it easier for the individual to find the optimal value of the current dimension, thus speeding up the convergence of the algorithm.
(2) Novel reinforcement of parent individual *X*_*p*2_
Unlike the parent individual *X*_*p*1_, which focuses on determining the evolutionary direction of the algorithm and improving the overall convergence speed, the parent individual *X*_*p*2_ focuses on providing excellent evolutionary information to guide the evolution of juveniles while maintaining population diversity. Given this, for the parent individual *X*_*p*2_, let it learn from the optimal individual *X*_*p*1_ and other individuals in the population together and propose a novel reinforcement approach as shown in Equation .
  (25) $$\begin{array}{c} X_{p2,j}\left(t\right)=X_{p2,j}\left(t-1\right)+r1\times \left(X_{p1,j}\left(t-1\right)-X_{p2,j}\left(t-1\right)\right)+G_{2}\times \left(X_{p2,j}\left(t-1\right)-X_{q,j}\left(t\right)\right), \end{array}$$
where individual *X*_*q*_ is a juvenile randomly selected from the population of juvenile crows after reinforcement learning, and *G*_2_ is a number that fits the Gaussian distribution *N*∼(*X*_*p*2,*j*_ (*t* − 1),0.5), as shown in Equation .
  (26) $$\begin{array}{c} G_{2}=\frac{1}{\sqrt{2\pi \times 0.5}}\times e^{-{\left(mean\left(j\right)-X_{p1,j}\left(t-1\right)\right)}^{2}/2\times 0.5}. \end{array}$$
Compared with the parent individual *X*_*p*1_ reinforcement method, the parent individual *X*_*p*2_ learns from the optimal individual *X*_*p*1_ when performing reinforcement to ensure that it does not deviate from the optimal evolutionary direction, but when referring to the evolutionary information of other individuals, it can explore in a more extensive search range, potentially providing information on other excellent locations that are not in the same region as the parent individual, making it possible for the juvenile individuals learning from it to explore in other regions that are not the same as *X*_*p*1_, further balancing the exploration and exploitation capabilities of the algorithm. In addition, the parent individual *X*_*p*2_ controls the scope of learning from the optimal individual *X*_*p*1_ and individual *X*_*q*_ with *r*1 and *G*_2_, respectively. In the early evolutionary stage, *G*_2_ is greater than r1 with a greater probability, i.e., compared with learning from the optimal individual, the parent individual *X*_*p*2_ learns more from the remaining individuals, which can better maintain population diversity, ensure the global search of the algorithm, and increase the possibility of convergence of the algorithm to the global optimum. In the late evolutionary stage, *G*_2_ is smaller than *r*1 with a greater probability, i.e., the parent individual *X*_*p*2_ learns mainly from the optimal individual, and learns supplementally from the rest of the individuals, further ensuring that individuals perform a refined search near the optimal individual, thus locking the global optimal position.

### 3.4. Algorithm Complexity Analysis

Assuming that the population size is *N*, the maximum number of iterations is *T*, the problem dimension is *D*, and the numbers of parent and juvenile jays are *N*_*P*_ and *N*_*J*_, respectively. The INCCLA algorithm mainly consists of the juvenile crow learning phase (*T*_*JL*_), the juvenile crow reinforcement phase (*T*_*JR*_), and the parent reinforcement phase (*T*_*PR*_). The worst time complexity of each stage of the INCCLA algorithm in a single run is analyzed as follows: in the juvenile crow learning stage (*T*_*JL*_), at most (*N*_*J*_ − *R*) × *N* times (1) needs to be computed, then the worst time complexity of this stage is *O* ((*N*_*J*_ − *R*) × *N*); in the juvenile crow reinforcement stage (*T*_*JR*_), at most *N*_*J*_ × *D* times (5) needs to be computed, then the worst time complexity of this stage is *O* (*N*_*J*_ × *D*); in the parent reinforcement stage (*T*_*PR*_), at most *N*_*P*_ × *D* times (23) or (25) needs to be computed, then the worst time complexity of this stage is *O* (*N*_*P*_ × *D*).

Therefore, the worst time complexity required for a single run of INCCLA is *O* ((*N*_*J*_ − *R*) × *N*) + *O* (*N*_*J*_ × *D*) + *O* (*N*_*P*_ × *D*) ≈ *O* (*T* × *N* × (*N*_*J*_ − *R* + *D*)).

## 4. Experimental Results and Discussion

In this section, to verify the performance of the INCCLA algorithm, the following four parts of experiments will be conducted in this paper: (1) The parameter sensitivity analysis; (2) Verification of the effectiveness of the proposed three improvement strategies; (3) Compare the performance of the improved INCCLA algorithm with the original NCCLA algorithm and four other representative and excellent performance evolutionary algorithms; (4) Comparison of the effectiveness of each algorithm in engineering applications.

This section uses the CEC2013 and CEC2020 test suites for experimental simulation. The CEC2013 test suite contains a total of 28 test functions, among which *F*1∼*F*5 are unimodal functions, which have only one optimal value and are used to verify the convergence performance of the algorithm; *F*6∼*F*20 are multimodal functions, which have multiple locally optimal solutions and are used to verify the ability of the algorithm to escape from the local optimum; *F*21∼*F*28 are composition functions. The CEC2020 test suite contains a total of 10 test functions, of which *F*1 is a unimodal function, *F*2∼*F*4 are multimodal shifted and rotated functions, *F*5∼*F*7 are hybrid functions, and *F*8∼*F*10 are composition functions. The relevant functions for the CEC2013 and CEC2020 test suites can be found in the literature [32, 33], respectively.

In this section, to ensure the fairness of the algorithm comparison, all algorithms were run on a computer with Windows 11 operating system, i5-11400H CPU, and programmed with MATLAB R2021a.

### 4.1. Sensitivity Analysis of Parameters

The INCCLA algorithm proposed in this paper involves five parameters: RP_prob_, SL_prob_, *R*, lf_min_, and lf_max_. Compared with the NCCLA algorithm, the INCCLA algorithm retains the originally proposed settings of RP_prob_ and SL_prob_, changes the settings of lf_min_ and lf_max_, and adds the parameter *R*. Given this, to analyze further the effect of parameters on the performance of the INCCLA algorithm, this section only analyzes the effect of parameters *R*, lf_min_ and lf_max_ on the performance of the INCCLA algorithm. To ensure fairness of comparison, the population size in each algorithm is *N* = 50, the dimension of the test function is *D* = 30, and the maximum number of function evaluations is MaxFEs = 150,000, RP_prob_ = 0.9, SL_prob_ = 0.99.

Table 1 gives the mean and average values of the optimal results obtained from 30 independent runs of the INCCLA algorithm on the CEC2013 test set when *R* is set to different parameters. In this experiment, lf_min_ = 0.0001 and lf_max_ = 0.09.  Table 2 give the mean and average values of the optimal results of the INCCLA algorithm for 30 independent runs on the CEC2013 test set when lf_min_ and lf_max_ are set to different combinations of parameters. For this experiment, *R* = 15. Tables 1 and 2 blacken the parameters that achieved the best results on each function and count the number of functions that performed best on each parameter set in the last row.

According to the data in Table 1, it can be seen that INCCLA achieves the best convergence on 19 test functions when *R* = 15. When *R* = 5, 25, and 35, the best convergence is achieved on 9, 11, and 14 test functions, respectively. Thus, the performance of INCCLA is sensitive to the setting of the parameter *R*, and the algorithm performs best when *R* = 15. Similarly, according to the data in Table 2, the performance of INCCLA is also sensitive to the settings of lf_min_ and lf_max_, and INCCLA achieves the best convergence among the 19 tested functions when lf_min_ = 0.0001 and lf_max_ = 0.09. In summary, if there is no special requirement, INCCLA with *R*, lf_min_, and lf_max_ set to 15, 0.0001, and 0.09, respectively, the algorithm can obtain better optimization results.

### 4.2. Experiment on Effectiveness of Each Improvement Strategy

According to Section 3, it is known that the INCCLA algorithm improves the NCCLA algorithm in three aspects. In this paper, to verify the effectiveness of the three improvement strategies, the NCCLA algorithm is combined with the three improvement strategies individually to form three new algorithms, namely, the INCCLA algorithm based on cosine similarity, the INCCLA algorithm based on improved juvenile learning phase, and the INCCLA algorithm based on improved reinforcement phase, named as INCCLA1, INCCLA2, and INCCLA3, respectively, and compared with the original NCCLA algorithm on the CEC2013 test suit.

In this section, to ensure fairness of comparison, the population size in each algorithm is *N* = 50, the dimension of the test function is *D* = 30, and the maximum number of function evaluations is MaxFEs = 5000 × *D* = 150,000. The other parameters of each algorithm are set as shown in Table 3. To avoid the contingency of a single operation of the algorithms, each algorithm was run 30 times independently on each test function.

Table 4 presents the running results of each algorithm on 28 test functions in 30 dimensions, where the “±” before and after represents the mean and standard deviation of the optimal values in 30 experiments, respectively, and the data that outperform the original NCCLA algorithm on the same function are marked in bold. To compare the significance of the performance of each improved strategy with the performance of NCCLA and to verify that the obtained results are not coincidental, Tables 5 and 6 present the results of the Wilcoxon rank sum test and Friedman test [34] between each improved strategy and NCCLA algorithm on 28 test functions, respectively. In Table 5, when the *p* value is greater than 0.05, it indicates that there is no significant difference between the improvement strategy and NCCLA, which is indicated by the symbol “ = .” When the *p* value is less than 0.05, and the mean value of the optimal solution of the result obtained in 30 experiments of the improvement strategy is better than NCCLA, it indicates that the improvement strategy is significantly better than NCCLA, which is indicated by the symbol “+”; otherwise, it indicates that the performance of the improvement strategy is significantly worse than NCCLA, which is indicated by the symbol “−.” In Table 6, the smaller the rank mean value corresponding to the algorithm, the better the algorithm's overall performance.

Table 4 shows that INCCLA1 obtains better mean values on all the remaining 24 test functions except *F*1, *F*8, *F*20, and *F*21 compared to NCCLA. INCCLA2 obtained better mean values on all 24 tested functions except *F*4, *F*8, *F*15, and F23; INCCLA3 obtained better mean values on all 26 tested functions except *F*17 and *F*27. As can be seen from Table 5, the Wilcoxon rank sum test results for INCCLA1 and NCCLA on the four tested functions of *F*4, *F*5, *F*10, and *F*13 are “+,” indicating that INCCLA1 outperforms NCCLA on these four functions. The Wilcoxon rank sum test result of “−” on the *F*21 test function indicates the inferior performance of INCCLA1 over NCCLA on *F*21, while the Wilcoxon rank sum test result of “ = ” on the remaining 23 test functions indicates that they perform similarly; INCCLA2 outperforms NCCLA on 14 test functions, has similar performance to NCCLA on 13 test functions, and inferior performance to NCCLA on F23 test functions; while INCCLA3 outperforms NCCLA on 15 test functions and has similar performance to NCCLA on 13 test functions. As can be seen from Table 6, the rank means of INCCLA2 is the smallest, indicating that the overall performance of the algorithm is superior, and the rank means of both INCCLA1 and INCCLA2 are smaller than those of NCCLA, indicating that all three improvement strategies proposed in this paper achieve better results.

In summary, all three improvement strategies proposed in this paper have certain improvement effects on NCCLA. The improvement strategies in the juvenile learning phase and the improvement strategies in the reinforcement phase have the most obvious improvement effects.

### 4.3. Performance Comparison of INCCLA with Other Algorithms

In this section, to verify the superior performance of the INCCLA algorithm in terms of convergence precision and convergence speed, this section compares the INCCLA with the NCCLA algorithm and the four better evolutionary algorithms on the CEC2013 and CEC2020 test suites, including the artificial bee colony algorithm based on new neighborhood selection mechanism (NSABC) [35], the sine cosine algorithm based on transition parameters and mutation operators (MSCA) [36], artificial tree algorithm based on two populations (IATTP) [37] and the improved crow search algorithm (ICSA) [38]. To ensure the fairness of the comparison, the population size in each algorithm is *N* = 50, and the maximum number of function evaluations is MaxFEs = 150,000. The other parameters of each algorithm are set as shown in Table 7, where the parameter values of each comparison algorithm are taken as in the original paper.

#### 4.3.1. Comparison of INCCLA with Other Algorithms on Convergence Precision

*(1) Testing at CEC 2013*. In order to fully compare the performance of INCCLA with other algorithms in terms of convergence precision, tests were conducted on the CEC2013 test suite with three different dimensions, *D* = 10, *D* = 30, and *D* = 100, respectively. Tables 8–10 give the mean and standard deviation of 30 independent experiments for each algorithm on the 10-dimension, 30-dimension, and 100-dimension CEC2013 datasets. The functions that achieved the best optimization results on the same functions are bold. To further verify the differences between INCCLA and each algorithm, the Wilcoxon rank sum test with a 5% significance level was performed between INCCLA and each algorithm, and the results are shown in Table 11. To comprehensively evaluate the overall performance of all algorithms, the results of the Friedman test are given in Table 12.

For the 10-dimensional optimization problem, as shown in Table 8, INCCLA achieves better mean values in all 28 test functions compared with NCCLA, and INCCLA achieves global optimum on 9 test functions, including *F*1, *F*3, *F*5, *F*7, *F*9, *F*11, *F*12, *F*13, and *F*20. Both the INCCLA algorithm and NSABC achieved the global optimum on nine test functions, including *F*1, *F*3, *F*5, *F*7, *F*9, *F*11, *F*12, *F*13, and *F*20, and the two algorithms achieved comparable mean values on functions F25 and *F*26. On five functions, including *F*19, *F*21, *F*24, *F*26, and *F*28, the INCCLA algorithm had inferior mean values to NSABC, and on the remaining 12 functions, the INCCLA algorithm obtained better mean values than NSABC. MSCA, IATTP, and ICSA all achieved theoretical optima on only seven test functions, including *F*3, *F*7, *F*9, *F*11, *F*12, *F*13, and *F*20. As seen in Table 11, NCCLA has similar performance on 10 functions compared to INCCLA, but significantly inferior performance on the 18 tested functions; NSABC performs significantly better on 4 functions but significantly inferior on 10 functions; MSCA has similar performance on 9 of the tested functions, but significantly inferior performance on the remaining 19 tested functions; IATTP has significantly better performance on *F*4, *F*26, and *F*27 only, but significantly inferior performance on the 14 tested functions; ICSA has significantly better performance on *F*26 only, but significantly inferior performance on all 14 functions. In summary, it shows that for low-dimensional optimization problems, the INCCLA proposed in this paper has some advantages in terms of convergence precision compared with other representative methods.

For the 30-dimensional optimization problem, it can be seen from Table 9 that INCCLA achieves the global optimum on nine test functions, including *F*1, *F*3, *F*5, *F*7, *F*9, *F*11, *F*12, *F*13, and *F*20. Like INCCLA, NCCLA also achieves the global optimum on these nine test functions, and INCCLA achieves worse mean values than NCCLA only on *F*4, but better mean values on the remaining test functions; NSABC achieved theoretical optima on six functions, including *F*1, *F*3, *F*5, *F*7, *F*9, and *F*11; MSCA obtained the theoretical optimal results on *F*3 and *F*11 only; IATTP obtained the theoretical optimal for six functions, including *F*3, *F*7, *F*9, *F*11, *F*12, and *F*13; ICSA obtained the theoretical optimal for five functions, including *F*3, *F*7, *F*9, *F*12, and *F*13. As seen in Table 11, compared to INCCLA, NCCLA has similar performance on 5 functions and significantly better performance on *F*4 only, but significantly inferior performance on the 22 tested functions; NSABC has significantly better performance on *F*6 and *F*26, but significantly inferior performance on 14 functions; MSCA has similar performance on 4 tested functions, but significantly inferior performance on the remaining 24 tested functions; IATTP had significantly better performance on *F*4 only, but significantly inferior performance on 17 test functions; ICSA has similar performance on 7 test functions only, but significantly inferior performance on the remaining 21 test functions. In summary, it shows that for the 30-dimensional CEC2013 test suite, the INCCLA proposed in this paper has a significant advantage in convergence accuracy compared with other representative methods, and the performance gap between algorithms is significantly more significant than that of the 10-dimensional optimization problem.

For the 100-dimensional optimization problem, it can be seen from Table 10 that INCCLA achieves the global optimum on three test functions, including *F*3, *F*7, and *F*11. NCCLA achieves the global optimum on *F*3 and *F*11, except that INCCLA and NCCLA obtain the same mean value on F8, NCCLA obtains a better mean value than INCCLA on *F*4, *F*14, *F*17, and *F*22, but NCCLA obtains a worse mean value than INCCLA on the rest of the 21 functions; NSABC obtained the global optimum on *F*3 and *F*11; MSCA obtained the theoretical optimum on *F*11 only; neither IATTP nor ICSA obtained the theoretical optimum on any function. As seen in Table 11, NCCLA performs significantly better on only four functions compared to INCCLA, including *F*4, *F*14, *F*17, and *F*22, but performs significantly inferior on the 20 test functions; NSABC has similar performance on 5 tested functions, significantly better performance on 7 functions, but significantly inferior performance on 16 functions; MSCA has similar performance on *F*8 and *F*11, but significantly inferior performance on the remaining 26 test functions; IATTP has significantly better performance on *F*4 only, but significantly inferior performance on the 24 test functions; ICSA has significantly better performance on *F*4 only, but significantly inferior performance on the 23 test functions. In summary, it shows that for high-dimensional optimization problems, the INCCLA proposed in this paper has a significant advantage in convergence precision compared with other representative methods, and the performance gap between the algorithms is more significant than that for optimization problems in 10 and 30 dimensions.

Table 12 shows that the overall performance of INCCLA is the best among the six optimization algorithms for the 10-dimensional, 30-dimensional, and 100-dimensional test functions, and its advantage is more obvious as the dimensionality of the optimization problem increases. In both 10-dimensional and 30-dimensional test functions, NSABC ranks second in overall performance, and IATTP, ICSA, and NCCLA are slightly worse than NSABC in both dimensions. In the 100-dimensional test function, the overall performance of NCCLA ranked second, and NSABC, ICSA, and IATTP were slightly worse than NCCLA in this dimension. The overall performance of MSCA was the worst among the six algorithms. In summary, compared with other algorithms, the INCCLA proposed in this paper has certain advantages in terms of convergence precision.

*(2) Testing at CEC 2020*. To further examine the performance of the INCCLA algorithm, the INCCLA algorithm and four other algorithms are tested on the 10-dimensional CEC2020 test suite. The parameters of each algorithm were set as above.  Table 13 counts the results of 30 independent experiments for each algorithm, including the mean and standard deviation, the results of the Wilcoxon rank sum test results for each algorithm with a significance level of 5% with the INCCLA algorithm, the number of functions for which each algorithm is significantly better than INCCLA, significantly worse than INCCLA, and not significantly different from INCCLA, and the results of the Fridman test and ranking results for each algorithm.

As shown in Table 13, for the 10-dimensional CEC2020 test function set, compared with NCCLA, INCCLA showed similar performance only on *F*10, achieved better mean values on the remaining 9 test functions, and performed significantly better on them. Compared with NSABC, INCCLA performs significantly inferior only on *F*9 and *F*3, achieves similar performance on 5 test functions, and performs significantly better on 3 test functions; compared to MSCA, INCCLA achieves better mean values on all 10 tested functions as well as showing significantly better performance. Compared to IATTP, INCCLA only showed inferior performance on *F*6 and *F*9, similar performance on *F*10, and significantly better performance on 7 test functions; compared to ICSA, INCCLA only showed inferior performance on *F*9, similar performance on *F*2 and *F*3, and significantly better performance on 7 test functions. It is obvious from the rank sum calibration results that INCCLA has an advantage over several other comparative algorithms on the CEC2020 test suite.

In summary, compared with NCCLA and the other four superior optimization algorithms, INCCLA shows a significant advantage in convergence precision. The advantages become more obvious as the dimension of the optimization problem increases.

#### 4.3.2. Comparison of INCCLA with Other Algorithms on Convergence Speed

In order to compare the differences in convergence speed among the algorithms more intuitively, Figure 4 shows the convergence curves of each algorithm on the 28 test functions of the CEC2013 test suite when the dimension is 30, where the horizontal coordinate is the number of function evaluations and the vertical coordinate is the logarithm of the fitness value.

As shown in Figure 4, for the unimodal functions *F*1∼*F*5, INCCLA can obtain the global optimum on *F*1, *F*3, and *F*5 test functions, but the convergence speed is slightly slower than NSABC on *F*1 and *F*5 test functions; INCCLA shows better convergence precision and the fastest convergence speed than the other five algorithms on *F*2; INCCLA is second only to IATTP in terms of convergence precision and convergence speed on *F*4. For multimodal functions *F*6∼*F*20, INCCLA can obtain the global optimum on *F*7, *F*9, *F*11, *F*12, *F*13, and *F*20 test functions, and the convergence speed is second only to MSCA on *F*11; INCCLA shows better convergence precision and the fastest convergence speed than the other five algorithms on *F*6, *F*10, and *F*19. INCCLA shows better convergence precision and relatively better convergence speed on *F*8, *F*14, *F*15, *F*16, *F*17, and *F*18 test functions. In the early evolutionary stage, the convergence speed of INCCLA is slightly slower than the other algorithms. When it reaches the late evolutionary stage, INCCLA can continue searching for better solutions compared to the reduced search performance of the other algorithms. For the composition functions *F*21∼*F*28, INCCLA shows better convergence precision and fastest convergence speed than the other five algorithms on the test functions *F*25, *F*27, and *F*28; INCCLA shows higher convergence precision and relatively faster convergence speed on *F*22 and *F*23. The convergence speed of INCCLA on *F*21 is similar to that of the three algorithms NSABC, NCCLA and IATTP, where the convergence precision of INCCLA and NSABC is slightly better than that of the other algorithms; the convergence speed of INCCLA on *F*24 is similar to that of the four algorithms NCCLA, ICSA, IATTP, and NSABC, with the convergence precision of INCCLA being higher. On *F*26, the convergence speed and precision of INCCLA are similar to those of ICSA and IATTP, and the convergence precision of INCCLA is second only to that of NSABC. In summary, it shows that INCCLA has some advantages in terms of convergence speed compared with NCCLA and the other four superior optimization algorithms.

In summary, compared with NCCLA and the other four superior optimization algorithms, the INCCLA proposed in this paper is superior in the overall performance in terms of convergence precision and convergence speed, although it has the shortcoming of not converging fast enough in the early stage for individual complex functions. The essential reasons for this are all caused by the three improved evolutionary strategies in Sections 3.1–3.3 of this paper, which are analyzed in depth as follows. The update strategy of the INCCLA algorithm has a large step size in the early evolutionary stage, which makes individuals search a farther distance around themselves, thus ensuring the global search of the algorithm and reducing the possibility of the algorithm falling into a local optimum, for more complex optimization problems, which also inevitably slows down the rapid aggregation of the population around a dominant region. Therefore, it makes INCCLA not converge fast enough in the early stage on individual complex functions. However, as the iteration proceeds, the individual search step size gradually decreases, and it is easier to search to have the advantage of the area, easy to refine the search, which improves the convergence speed in the late evolutionary stage and facilitates the algorithm to obtain a more excellent convergence precision. In addition, the parental selection mechanism can guide the evolutionary direction of juveniles during the learning phase, allowing the algorithm to increase algorithmic diversity while maintaining convergence. The juvenile crow hybrid learning mechanism can determine the state of the algorithm in the current evolutionary stage according to the individual's attributes and select the learning mode in a targeted manner so that the algorithm can effectively maintain the balance of convergence speed and diversity in the evolutionary process. The interplay and influence of these three mechanisms ensures the overall advantage of INCCLA in terms of convergence precision and convergence speed. In the next step, we will work on further improving the convergence speed of the INCCLA algorithm in the pre-evolutionary stage while ensuring no significant change in the convergence precision.

### 4.4. Comparison of the Effects of Engineering Applications

To further compare the effectiveness of INCCLA with each comparison algorithm for engineering applications, this section will be validated by dealing with the collaborative beamforming optimization problem. The collaborative beamforming optimization problem is a typical problem in antenna arrays. The amplitude *ξ* ∈ [0,1] and phase *α* ∈ [−*π *, *π*] of the transmit signal weights of each collaborative node are used as decision variables in the algorithm optimization process, and the peak side valve level PSL minimization as shown in (27) is achieved by algorithm optimization.

(27) $$\begin{array}{c} PSL=20\;\log_{10}\frac{\max\left|AF\left(\theta_{SL},w\right)\right|}{AF\left(\phi ,w\right)}, \end{array}$$

where, AF(*θ*, *w*) represents the array factor, as shown in (28) and *φ* is the main beam direction. The positions of *θ*_*SL*_ can be found by finding all the peak points of the array factor (other than the main lobe's peak) for the domain *θ* ∈ [−*π*, *ϕ*) ∪ (*ϕ*, *π*], the denominator *AF*(*ϕ*, *w*) is the main beam power, which can be calculated as described in the literature [39], and molecule max|*AF*(*θ*_*SL*_, *w*)| is the maximum beam power in the side flap.

(28) $$\begin{array}{c} AF\left(\theta ,w\right)=\sum_{k=1}^{k}w_{k}e^{j\left(2\pi /\lambda \right)r_{k}\left[\cos\left(\theta -\psi_{k}\right)\right]}. \end{array}$$

This section examines the practical engineering optimization of INCCLA and the other comparative algorithms by optimizing the collaborative beamforming problem shown in Figure 5, in which the wavelength of the transmitting signal is *λ*. The six synergistic nodes are distributed in a circular domain of radius 6*λ*, where one synergistic node is located in the center of the circular domain.

The parameter settings of each algorithm are shown in Table 7. In order to avoid adverse effects of chance on algorithm evaluation, each algorithm was run 10 times independently. The best median PSL obtained by each algorithm corresponding to the collaborative beam optimization scheme was selected for comparison. The beam diagram of INCCLA with each comparison algorithm in the Cartesian coordinate system is visually presented in Figure 6. The PSL obtained by each algorithm is labeled within the figure.

According to Figure 6, it can be seen that each algorithm achieves better collaborative beam optimization compared to the unoptimized algorithm, where the best PSL values obtained by INCCLA, NCCLA, NSABC, MSCA, IATTP, and ICSA are −5.5044 dB, −5.2306 dB, −5.2181 dB, −3.5948 dB, −4.1655 dB, and −5.3668 dB, respectively. Compared with the other five algorithms, the best PSL value obtained by INCCLA is the smallest and achieves the best collaborative beam optimization among the five algorithms. In summary, the proposed INCCLA also performs better in engineering applications.

## 5. Conclusions

This paper proposes an improved New Caledonian Crow Learning Algorithm (INCCLA) to improve further the convergence performance and the ability to escape from the local optimum of the NCCLA algorithm. First, INCCLA introduces cosine similarity in the parent selection phase. The selected parent can guide the juvenile crow to exploit different regions, maintaining the balance between population diversity and the convergence speed of the algorithm in the evolutionary process. Second, INCCLA sets up a mixed learning mechanism of complete learning and incomplete learning, with the complete learning phase accelerating individual convergence and improving the convergence speed of the algorithm, and the incomplete learning phase increasing population diversity and enhancing the ability of the algorithm to escape from the local optimum. Finally, the juvenile crow reinforcement phase introduces weight factors and random perturbations to increase the global search and local exploration ability of the algorithm in the evolutionary process. The proposed parent reinforcement phase enhances the individual search capability of the parent and improves the overall performance of the algorithm. Experimental results on the CEC2013 and CEC2020 test suites show that the improvement strategy proposed in this paper effectively improves the overall performance of INCCLA, enabling the algorithm to maintain a balance between convergence speed and population diversity during the evolutionary process, and can achieve better results in most of the test functions. In addition, INCCLA is also more competitive in unimodal, multimodal, and composition problems compared with the other four optimization algorithms. INCCLA is also applied to the collaborative beamforming optimization problem, demonstrating the usefulness of INCCLA in engineering applications.

Although the INCCLA algorithm proposed in this paper has obvious advantages in terms of convergence accuracy, its time complexity is slightly higher. In future work, the time complexity of the algorithm needs to be further reduced. In addition, it further broadens the application of the INCCLA algorithm in practical engineering fields.

## Figures and Tables

**Figure 1:** Schematic of the process of determining parent individuals based on cosine similarity.

**Figure 2:** Schematic of juvenile crow learning phase.

**Figure 3:** Schematic diagram of the variation of weighting factors with iterations.

**Figure 4:** Convergence curves of each algorithm on the CEC2013 test suite. (a)-(ab) denote the 28 test functions *F*1∼*F*28 in the CEC2013 test set, respectively.

**Figure 5:** Distribution of synergy nodes.

**Figure 6:** Beam diagram of INCCLA and each comparison algorithm in the cartesian coordinate system. (a)–(e) are the beam diagram of INCCLA with NCCLA, NSABC, MSCA, IATTP, and ICSA, respectively.

**Algorithm 1:** NCCLA.

**Algorithm 2:** INCCLA.

**Table 1:** Effect of parameter *R* on the performance of the algorithm.

Function	*R* = 5	*R* = 15	*R* = 25	*R* = 35
F1	**0.00E** **+** **00** **±** **0.00E** **+** **00**	**0.00E** **+** **00** **±** **0.00E** **+** **00**	**0.00E** **+** **00** **±** **0.00E** **+** **00**	**0.00E** **+** **00** **±** **0.00E** **+** **00**
F2	**7.62E** **+** **05** **±** **3.02E** **+** **05**	8.10*E* **+** 05 **±** 4.96*E* **+** 05	7.76*E* **+** 05 **±** 3.66*E* **+** 05	2.45*E* **+** 06 **±** 3.89*E* **+** 06
F3	**0.00E** **+** **00** **±** **0.00E** **+** **00**	**0.00E** **+** **00** **±** **0.00E** **+** **00**	**0.00E** **+** **00** **±** **0.00E** **+** **00**	**0.00E** **+** **00** **±** **0.00E** **+** **00**
F4	1.13*E* **+** 04 **±** 3.87*E* **+** 03	**1.10E** **+** **04** **±** **3.46E** **+** **03**	1.43*E* **+** 04 **±** 3.64*E* **+** 03	1.82*E* **+** 04 **±** 4.62*E* **+** 03
F5	**0.00E** **+** **00** **±** **0.00E** **+** **00**	**0.00E** **+** **00** **±** **0.00E** **+** **00**	**0.00E** **+** **00** **±** **0.00E** **+** **00**	**0.00E** **+** **00** **±** **0.00E** **+** **00**
F6	2.87*E* **+** 01 **±** 2.49*E* **+** 01	**2.40E** **+** **01** **±** **2.04E** **+** **01**	2.91*E* **+** 01 **±** 2.50*E* **+** 01	3.39*E* **+** 01 **±** 2.58*E* **+** 01
F7	**0.00E** **+** **00** **±** **0.00E** **+** **00**	**0.00E** **+** **00** **±** **0.00E** **+** **00**	**0.00E** **+** **00** **±** **0.00E** **+** **00**	**0.00E** **+** **00** **±** **0.00E** **+** **00**
F8	**2.09E** **+** **01** **±** **4.40E** − **02**	2.10*E* **+** 01 **±** 5.23*E* − 02	2.09*E* **+** 01 **±** 8.22*E* − 02	2.10*E* **+** 01 **±** 5.06*E* − 02
F9	**0.00E** **+** **00** **±** **0.00E** **+** **00**	**0.00E** **+** **00** **±** **0.00E** **+** **00**	**0.00E** **+** **00** **±** **0.00E** **+** **00**	**0.00E** **+** **00** **±** **0.00E** **+** **00**
F10	2.68*E* − 01 **±** 9.36*E* − 02	2.10*E* − 01 **±** 5.91*E* − 02	1.91*E* − 01 **±** 7.21*E* − 02	**1.24E** − **01** **±** **5.80E** − **02**
F11	**0.00E** **+** **00** **±** **0.00E** **+** **00**	**0.00E** **+** **00** **±** **0.00E** **+** **00**	**0.00E** **+** **00** **±** **0.00E** **+** **00**	**0.00E** **+** **00** **±** **0.00E** **+** **00**
F12	4.00*E* **+** 00 **±** 2.15*E* **+** 01	**0.00E** **+** **00** **±** **0.00E** **+** **00**	4.08*E* **+** 00 **±** 2.23*E* **+** 01	**0.00E** **+** **00** **±** **0.00E** **+** **00**
F13	4.86*E* **+** 00 **±** 2.62*E* **+** 01	**0.00E** **+** **00** **±** **0.00E** **+** **00**	**0.00E** **+** **00** **±** **0.00E** **+** **00**	**0.00E** **+** **00** **±** **0.00E** **+** **00**
F14	6.82*E* **+** 00 **±** 4.57*E* **+** 00	**6.29E** **+** **00** **±** **4.92E** **+** **00**	3.88*E* **+** 01 **±** 7.61*E* **+** 01	5.26*E* **+** 01 **±** 7.95*E* **+** 01
F15	4.07*E* **+** 03 **±** 5.73*E* **+** 02	3.94*E* **+** 03 **±** 6.65*E* **+** 02	**3.69E** **+** **03** **±** **4.42E** **+** **02**	3.69*E* **+** 03 **±** 7.34*E* **+** 02
F16	1.03*E* **+** 00 **±** 3.89*E* − 01	**9.33E** − **01** **±** **2.63E** − **01**	9.36*E* − 01 **±** 3.55*E* − 01	9.57*E* − 01 **±** 2.58*E* − 01
F17	4.28*E* **+** 00 **±** 7.40*E* **+** 00	**5.43E** **+** **00** **±** **7.92E** **+** **00**	7.20*E* **+** 00 **±** 9.07*E* **+** 00	8.64*E* **+** 00 **±** 4.20*E* **+** 00
F18	1.18*E* **+** 02 **±** 3.47*E* **+** 01	9.65*E* **+** 01 **±** 2.06*E* **+** 01	9.90*E* **+** 01 **±** 2.63*E* **+** 01	**8.60E** **+** **01** **±** **2.39E** **+** **01**
F19	6.73*E* **+** 00 **±** 1.85*E* **+** 00	**5.32E** **+** **00** **±** **2.09E** **+** **00**	5.42*E* **+** 00 **±** 1.54*E* **+** 00	5.53*E* **+** 00 **±** 1.84*E* **+** 00
F20	1.94*E* − 01 **±** 1.05*E* **+** 00	**0.00E** **+** **00** **±** **0.00E** **+** **00**	**0.00E** **+** **00** **±** **0.00E** **+** **00**	**0.00E** **+** **00** **±** **0.00E** **+** **00**
F21	4.15*E* **+** 02 **±** 8.03*E* **+** 01	**4.00E** **+** **02** **±** **0.00E** **+** **00**	**4.00E** **+** **02** **±** **0.00E** **+** **00**	**4.00E** **+** **02** **±** **0.00E** **+** **00**
F22	9.01*E* **+** 01 **±** 6.02*E* **+** 01	**7.70E** **+** **01** **±** **5.90E** **+** **01**	1.10*E* **+** 02 **±** 6.44*E* **+** 01	1.11*E* **+** 02 **±** 7.74*E* **+** 01
F23	3.96*E* **+** 03 **±** 5.75*E* **+** 02	4.06*E* **+** 03 **±** 5.45*E* **+** 02	**3.55E** **+** **03** **±** **7.00E** **+** **02**	3.67*E* **+** 03 **±** 6.44*E* **+** 02
F24	**2.00E** **+** **02** **±** **1.81E** − **02**	2.00*E* **+** 02 **±** 2.44*E* − 02	2.00*E* **+** 02 **±** 2.13*E* − 02	2.00*E* **+** 02 **±** 1.93*E* − 02
F25	2.59*E* **+** 02 **±** 3.90*E* **+** 01	2.40*E* **+** 02 **±** 3.15*E* **+** 01	2.42*E* **+** 02 **±** 3.21*E* **+** 01	**2.23E** **+** **02** **±** **2.13E** **+** **01**
F26	3.06*E* **+** 02 **±** 1.60*E* **+** 01	**2.87E** **+** **02** **±** **3.45E** **+** **01**	2.97*E* **+** 02 **±** 1.82*E* **+** 01	3.00*E* **+** 02 **±** 5.68*E* − 07
F27	3.27*E* **+** 02 **±** 7.05*E* **+** 01	**3.13E** **+** **02** **±** **8.90E** − **01**	3.13*E* **+** 02 **±** 9.46*E* − 01	3.13*E* **+** 02 **±** 9.22*E* − 01
F28	9.64*E* **+** 02 **±** 3.39*E* **+** 01	9.14*E* **+** 02 **±** 2.15*E* **+** 01	8.83*E* **+** 02 **±** 1.81*E* **+** 01	**8.60E** **+** **02** **±** **1.80E** **+** **01**
	9	19	11	14

Bold indicates the best results obtained on each function.

**Table 2:** Effect of parameters lf_min_ and lf_max_ on the performance of the algorithm.

Function	lf_min_ = 0.0001, lf_max_ = 0.005	lf_min_ = 0.0001, lf_max_ = 0.09	lf_min_ = 0.0005, lf_max_ = 0.02	lf_min_ = 0.005, lf_max_ = 0.2
F1	**0.00E** **+** **00** ± **0.00E** **+** **00**	**0.00E** **+** **00** ± **0.00E** **+** **00**	**0.00E** **+** **00** ± **0.00E** **+** **00**	**0.00E** **+** **00** ± **0.00E** **+** **00**
F2	1.03*E* **+** 06 ± 6.20*E* **+** 05	**8.10E** **+** **05** ± **4.96E** **+** **05**	8.62*E* **+** 05 ± 5.43*E* **+** 05	9.26*E* **+** 05 ± 5.10*E* **+** 05
F3	**0.00E** **+** **00** ± **0.00E** **+** **00**	**0.00E** **+** **00** ± **0.00E** **+** **00**	**0.00E** **+** **00** ± **0.00E** **+** **00**	**0.00E** **+** **00** ± **0.00E** **+** **00**
F4	1.42*E* **+** 04 ± 4.01*E* **+** 03	**1.10E** **+** **04** ± **3.46E** **+** **03**	1.25*E* **+** 04 ± 3.36*E* **+** 03	1.28*E* **+** 04 ± 3.47*E* **+** 03
F5	**0.00E** **+** **00** ± **0.00E** **+** **00**	**0.00E** **+** **00** ± **0.00E** **+** **00**	**0.00E** **+** **00** ± **0.00E** **+** **00**	**0.00E** **+** **00** ± **0.00E** **+** **00**
F6	2.99*E* **+** 01 ± 2.55*E* **+** 01	**2.40E** **+** **01** ± **2.04E** **+** **01**	2.61*E* **+** 01 ± 2.29*E* **+** 01	2.60*E* **+** 01 ± 2.23*E* **+** 01
F7	**0.00E** **+** **00** ± **0.00E** **+** **00**	**0.00E** **+** **00** ± **0.00E** **+** **00**	**0.00E** **+** **00** ± **0.00E** **+** **00**	**0.00E** **+** **00** ± **0.00E** **+** **00**
F8	2.10*E* **+** 01 ± 4.85*E* − 02	2.10*E* **+** 01 ± 5.23*E* − 02	**2.10E** **+** **01** ± **4.17E** − **02**	2.10*E* **+** 01 ± 5.84*E* − 02
F9	8.85*E* − 01 ± 4.85*E* **+** 00	**0.00E** **+** **00** ± **0.00E** **+** **00**	**0.00E** **+** **00** ± **0.00E** **+** **00**	**0.00E** **+** **00** ± **0.00E** **+** **00**
F10	2.12*E* − 01 ± 9.61*E* − 02	**2.10E** − **01** ± **5.91E** − **02**	2.16*E* − 01 ± 6.67*E* − 02	2.15*E* − 01 ± 7.12*E* − 02
F11	**0.00E** **+** **00** ± **0.00E** **+** **00**	**0.00E** **+** **00** ± **0.00E** **+** **00**	**0.00E** **+** **00** ± **0.00E** **+** **00**	**0.00E** **+** **00** ± **0.00E** **+** **00**
F12	**0.00E** **+** **00** ± **0.00E** **+** **00**	**0.00E** **+** **00** ± **0.00E** **+** **00**	**0.00E** **+** **00** ± **0.00E** **+** **00**	**0.00E** **+** **00** ± **0.00E** **+** **00**
F13	4.75*E* **+** 00 ± 2.60*E* **+** 01	**0.00E** **+** **00** ± **0.00E** **+** **00**	**0.00E** **+** **00** ± **0.00E** **+** **00**	**0.00E** **+** **00** ± **0.00E** **+** **00**
F14	6.81*E* **+** 02 ± 8.45*E* **+** 02	**6.29E** **+** **00** ± **4.92E** **+** **00**	1.38*E* **+** 02 ± 3.17*E* **+** 02	9.30*E* **+** 00 ± 2.29*E* **+** 01
F15	4.21*E* **+** 03 ± 5.84*E* **+** 02	3.94*E* **+** 03 ± 6.65*E* **+** 02	3.89*E* **+** 03 ± 7.58*E* **+** 02	**3.78E** **+** **03** ± **6.28E** **+** **02**
F16	1.02*E* **+** 00 ± 3.13*E* − 01	**9.33E** − **01** ± **2.63E** − **01**	9.73*E* − 01 ± 2.67*E* − 01	9.77*E* − 01 ± 3.63*E* − 01
F17	3.17*E* **+** 01 ± 4.06*E* **+** 01	5.43*E* **+** 00 ± 7.92*E* **+** 00	1.05*E* **+** 01 ± 1.10*E* **+** 01	**4.87E** **+** **00** ± **8.60E** **+** **00**
F18	1.29*E* **+** 02 ± 2.59*E* **+** 01	**9.65E** **+** **01** ± **2.06E** **+** **01**	1.19*E* **+** 02 ± 3.04*E* **+** 01	9.69*E* **+** 01 ± 2.65*E* **+** 01
F19	7.11*E* **+** 00 ± 2.59*E* **+** 00	5.32*E* **+** 00 ± 2.09*E* **+** 00	6.10*E* **+** 00 ± 2.32*E* **+** 00	**5.27E** **+** **00** ± **1.94E** **+** **00**
F20	2.72*E* − 01 ± 1.49*E* **+** 00	**0.00E** **+** **00** ± **0.00E** **+** **00**	**0.00E** **+** **00** ± **0.00E** **+** **00**	**0.00E** **+** **00** ± **0.00E** **+** **00**
F21	4.00*E* **+** 02 ± 0.00*E* **+** 00	4.00*E* **+** 02 ± 0.00*E* **+** 00	**3.93E** **+** **02** ± **3.65E** **+** **01**	4.00*E* **+** 02 ± 0.00*E* **+** 00
F22	5.18*E* **+** 02 ± 8.92*E* **+** 02	**7.70E** **+** **01** ± **5.90E** **+** **01**	1.25*E* **+** 02 ± 7.26*E* **+** 01	1.16*E* **+** 02 ± 5.89*E* **+** 01
F23	4.06*E* **+** 03 ± 7.22*E* **+** 02	4.06*E* **+** 03 ± 5.45*E* **+** 02	4.29*E* **+** 03 ± 6.34*E* **+** 02	**4.02E** **+** **03** ± **6.07E** **+** **02**
F24	2.00*E* **+** 02 ± 2.30*E* − 02	2.00*E* **+** 02 ± 2.44*E* − 02	**2.00E** **+** **02** ± **2.24E** − **02**	2.00*E* **+** 02 ± 2.46*E* − 02
F25	**2.34E** **+** **02** ± **3.04E** **+** **01**	2.40*E* **+** 02 ± 3.15*E* **+** 01	2.51*E* **+** 02 ± 3.59*E* **+** 01	2.56*E* **+** 02 ± 3.80*E* **+** 01
F26	3.01*E* **+** 02 ± 7.13*E* **+** 00	**2.87E** **+** **02** ± **3.45E** **+** **01**	2.97*E* **+** 02 ± 2.91*E* **+** 01	2.98*E* **+** 02 ± 2.03*E* **+** 01
F27	3.14*E* **+** 02 ± 1.49*E* **+** 00	**3.13E** **+** **02** ± **8.90E** − **01**	3.13*E* **+** 02 ± 1.03*E* **+** 00	3.13*E* **+** 02 ± 1.14*E* **+** 00
F28	9.10*E* **+** 02 ± 2.50*E* **+** 01	9.14*E* **+** 02 ± 2.15*E* **+** 01	**9.07E** **+** **02** ± **1.73E** **+** **01**	9.19*E* **+** 02 ± 2.33*E* **+** 01
	7	19	13	13

Bold indicates the best results obtained on each function.

**Table 3:** Algorithm-related parameters.

Algorithm	Parameter
NCCLA	RP_prob_ = 0.9; SL_prob_ = 0.99; VSL_prob_ = 0.99; P1_prob_ = 0.95; TaE_prob_ = 0.3; lf_min_ = 0.0005; lf_max_ = 0.02
INCCLA1	RP_prob_ = 0.9; SL_prob_ = 0.99; VSL_prob_ = 0.99; P1_prob_ = 0.95; TaE_prob_ = 0.3; lf_min_ = 0.0005; lf_max_ = 0.02
INCCLA2	RP_prob_ = 0.9; SL_prob_ = 0.99; R = 15; lf_min_ = 0.0005; lf_max_ = 0.02
INCCLA3	RP_prob_ = 0.9; SL_prob_ = 0.99; VSL_prob_ = 0.99; P1_prob_ = 0.95; TaE_prob_ = 0.3; lf_min_ = 0.0001; lf_max_ = 0.09

**Table 4:** Results of each improvement strategy in the 30-dimensional CEC2013 test suite.

Function	NCCLA	INCCLA1	INCCLA2	INCCLA3
*F*1	1.99*E* − 05 ± 5.60*E* − 05	4.22*E* − 05 ± 1.59*E* − 04	**4.19E** − **06** ± **1.30E** − **05**	**2.10E** − **30** ± **9.42E** − **30**
*F*2	7.59*E* **+** 06 ± 4.32*E* **+** 06	**6.38E** **+** **06** ± **3.75E** **+** **06**	**6.37E** **+** **06** ± **3.13E** **+** **06**	**7.13E** **+** **05** ± **2.69E** **+** **05**
*F*3	0.00*E* **+** 00 ± 0.00*E* **+** 00	**0.00E** **+** **00** ± **0.00E** **+** **00**	**0.00E** **+** **00** ± **0.00E** **+** **00**	**0.00E** **+** **00** ± **0.00E** **+** **00**
*F*4	7.59*E* **+** 03 ± 2.43*E* **+** 03	**6.33E** **+** **03** ± **2.47E** **+** **03**	8.13*E* **+** 03 ± 2.51*E* **+** 03	**3.28E** **+** **03** ± **1.98E** **+** **03**
*F*5	8.91*E* − 04 ± 3.77*E* − 03	**3.42E** − **05** ± **8.93E** − **05**	**6.86E** − **05** ± **2.37E** − **04**	**0.00E** **+** **00** ± **0.00E** **+** **00**
*F*6	6.64*E* **+** 01 ± 3.21*E* **+** 01	**5.82E** **+** **01** ± **2.90E** **+** **01**	**5.15E** **+** **01** ± **2.35E** **+** **01**	**3.12E** **+** **01** ± **2.78E** **+** **01**
*F*7	0.00*E* **+** 00 ± 0.00*E* **+** 00	**0.00E** **+** **00** ± **0.00E** **+** **00**	**0.00E** **+** **00** ± **0.00E** **+** **00**	**0.00E** **+** **00** ± **0.00E** **+** **00**
*F*8	2.10*E* **+** 01 ± 5.25*E* − 02	2.10*E* **+** 01 ± 5.42*E* − 02	**2.10E** **+** **01** ± **4.17E** − **02**	**2.10E** **+** **01** ± **3.49E** − **02**
*F*9	5.26*E* **+** 00 ± 9.82*E* **+** 00	**2.23E** **+** **00** ± **6.87E** **+** **00**	**0.00E** **+** **00** ± **0.00E** **+** **00**	**2.52E** **+** **00** ± **7.71E** **+** **00**
*F*10	9.26*E* **+** 00 ± 7.28*E* **+** 00	**6.80E** **+** **00** ± **5.65E** **+** **00**	**6.67E** **+** **00** ± **3.25E** **+** **00**	**2.16E** − **01** ± **1.98E** − **01**
*F*11	0.00*E* **+** 00 ± 0.00*E* **+** 00	**0.00E** **+** **00** ± **0.00E** **+** **00**	**0.00E** **+** **00** ± **0.00E** **+** **00**	**0.00E** **+** **00** ± **0.00E** **+** **00**
*F*12	1.16*E* **+** 02 ± 3.57*E* **+** 01	**8.96E** **+** **01** ± **6.22E** **+** **01**	**0.00E** **+** **00** ± **0.00E** **+** **00**	**1.02E** **+** **02** ± **7.05E** **+** **01**
*F*13	1.31*E* **+** 02 ± 6.87*E* **+** 01	**1.18E** **+** **02** ± **6.15E** **+** **01**	**0.00E** **+** **00** ± **0.00E** **+** **00**	**1.07E** **+** **02** ± **8.38E** **+** **01**
*F*14	1.78*E* **+** 01 ± 3.12*E* **+** 01	**8.96E** **+** **00** ± **4.34E** **+** **00**	**4.24E** **+** **00** ± **2.81E** **+** **00**	**1.15E** **+** **01** ± **2.49E** **+** **01**
*F*15	4.79*E* **+** 03 ± 1.50*E* **+** 03	**4.33E** **+** **03** ± **1.14E** **+** **03**	7.17*E* **+** 03 ± 2.72*E* **+** 02	**3.65E** **+** **03** ± **5.90E** **+** **02**
*F*16	2.68*E* **+** 00 ± 3.22*E* − 01	**2.50E** **+** **00** ± **3.43E** − **01**	**2.62E** **+** **00** ± **2.98E** − **01**	**1.06E** **+** **00** ± **3.87E** − **01**
*F*17	9.59*E* **+** 00 ± 1.21*E* **+** 01	**7.98E** **+** **00** ± **1.19E** **+** **01**	**5.44E** **+** **00** ± **6.87E** **+** **00**	1.10*E* **+** 01 ± 1.37*E* **+** 01
*F*18	1.77*E* **+** 02 ± 4.90*E* **+** 01	**1.66E** **+** **02** ± **4.61E** **+** **01**	**1.43E** **+** **02** ± **4.88E** **+** **01**	**1.54E** **+** **02** ± **3.64E** **+** **01**
*F*19	1.57*E* **+** 01 ± 7.70*E* **+** 00	**1.47E** **+** **01** ± **6.78E** **+** **00**	**7.74E** **+** **00** ± **2.36E** **+** **00**	**9.11E** **+** **00** ± **2.73E** **+** **00**
*F*20	1.31*E* **+** 01 ± 3.16*E* **+** 00	1.34*E* **+** 01 ± 2.31*E* **+** 00	**0.00E** **+** **00** ± **0.00E** **+** **00**	**1.20E** **+** **01** ± **3.58E** **+** **00**
*F*21	4.00*E* **+** 02 ± 2.73*E* − 01	4.00*E* **+** 02 ± 3.12*E* − 01	**4.00E** **+** **02** ± **1.97E** − **01**	**4.00E** **+** **02** ± **7.62E** − **12**
*F*22	1.17*E* **+** 02 ± 6.11*E* **+** 01	**7.99E** **+** **01** ± **7.61E** **+** **01**	**9.09E** **+** **01** ± **6.46E** **+** **01**	**1.04E** **+** **02** ± **8.25E** **+** **01**
*F*23	4.21*E* **+** 03 ± 6.46*E* **+** 02	**4.07E** **+** **03** ± **1.11E** **+** **03**	6.90*E* **+** 03 ± 4.60*E* **+** 02	**3.87E** **+** **03** ± **9.03E** **+** **02**
*F*24	2.04*E* **+** 02 ± 1.37*E* **+** 01	**2.01E** **+** **02** ± **7.70E** − **01**	**2.00E** **+** **02** ± **4.13E** − **02**	**2.02E** **+** **02** ± **1.10E** **+** **01**
*F*25	2.88*E* **+** 02 ± 3.40*E* **+** 01	**2.79E** **+** **02** ± **3.98E** **+** **01**	**2.48E** **+** **02** ± **4.21E** **+** **01**	**2.85E** **+** **02** ± **3.25E** **+** **01**
*F*26	3.08*E* **+** 02 ± 4.25*E* **+** 01	**2.99E** **+** **02** ± **4.17E** **+** **01**	**2.97E** **+** **02** ± **1.82E** **+** **01**	**2.97E** **+** **02** ± **3.89E** **+** **01**
*F*27	4.46*E* **+** 02 ± 2.75*E* **+** 02	**3.94E** **+** **02** ± **1.81E** **+** **02**	**3.22E** **+** **02** ± **2.68E** **+** **00**	6.16*E* **+** 02 ± 3.16*E* **+** 02
*F*28	1.46*E* **+** 03 ± 8.95*E* **+** 02	**1.21E** **+** **03** ± **5.33E** **+** **02**	**1.08E** **+** **03** ± **5.76E** **+** **01**	**1.05E** **+** **03** ± **3.53E** **+** **02**

Bold indicates the best results obtained on each function.

**Table 5:** Wilcoxon rank sum test results between NCCLA and each improvement strategy.

Function	*p* value (vs.NCCLA)		
	INCCLA1	INCCLA2	INCCLA3
*F*1	0.876 (=)	0.053 (=)	0.000 (+)
*F*2	0.304 (=)	0.379 (=)	0.000 (+)
*F*3	1.000 (=)	1.000 (=)	1.000 (=)
*F*4	0.029 (+)	0.363 (=)	0.000 (+)
*F*5	0.003 (+)	0.004 (+)	0.000 (+)
*F*6	0.559 (=)	0.082 (=)	0.000 (+)
*F*7	1.000 (=)	1.000 (=)	1.000 (=)
*F*8	0.067 (=)	0.340 (=)	0.077 (=)
*F*9	0.179 (=)	0.005 (+)	0.218 (=)
*F*10	0.035 (+)	0.270 (=)	0.000 (+)
*F*11	1.000 (=)	1.000 (=)	1.000 (=)
*F*12	0.302 (=)	0.000 (+)	0.385 (=)
*F*13	0.025 (+)	0.000 (+)	0.616 (=)
*F*14	0.491 (=)	0.000 (+)	0.012 (+)
*F*15	0.099 (=)	0.000 (+)	0.000 (+)
*F*16	0.057 (=)	0.395 (=)	0.000 (+)
*F*17	0.090 (=)	0.118 (=)	0.137 (=)
*F*18	0.420 (=)	0.006 (+)	0.045 (+)
*F*19	0.706 (=)	0.000 (+)	0.000 (+)
*F*20	0.264 (=)	0.000 (+)	0.273 (=)
*F*21	0.019 (-)	0.994 (=)	0.000 (+)
*F*22	0.067 (=)	0.050 (=)	0.911 (=)
*F*23	0.112 (=)	0.000 (-)	0.108 (=)
*F*24	0.482 (=)	0.000 (+)	0.000 (+)
*F*25	0.807 (=)	0.000 (+)	0.473 (=)
*F*26	0.529 (=)	0.000 (+)	0.000 (+)
*F*27	0.599 (=)	0.000 (+)	0.510 (=)
*F*28	0.258 (=)	0.002 (+)	0.000 (+)
+/=/−	4/23/1	14/13/1	15/13/0

**Table 6:** Friedman test results for four algorithms.

	NCCLA	INCCLA1	INCCLA2	INCCLA3
Avg.rank	3.48	2.48	1.96	2.07
Sort	4	3	1	2

**Table 7:** Related parameter settings of each algorithm.

Algorithm	Parameter
NCCLA	RP_prob_ = 0.9; SL_prob_ = 0.99; VSL_prob_ = 0.99; P1_prob_ = 0.95; TaE_prob_ = 0.3; lf_min_ = 0.0005; lf_max_ = 0.02
NSABC	*C* = 1.5; limit = 100; *k* = 10
MSCA	*a* = 2; *b* = 0.5
IATTTP	*h*1 = *h*2 = *h*3 = 0.5, *h*4 = 0.8, *m* = 50, *q* = 0.8
ICSA	*AP* = 0.1; *FL* = 1.5
INCCLA	RP_prob_ = 0.9; SL_prob_ = 0.99; *R* *=* *15*; lf_min_ = 0.0001; lf_max_ = 0.09

**Table 8:** Data result of INCCLA with other algorithms on the 10-dimensional CEC2013 test suite.

Fun.	NSABC		MSCA		IATTP		ICSA		NCCLA		INCCLA	
	Mean	Std	Mean	Std	Mean	Std	Mean	Std	Mean	Std	Mean	Std
*F*1	**0.00E + 00**	**0.00*E* + 00**	2.17*E* + 02	2.79*E* + 02	8.91*E* − 03	1.05*E* − 02	4.53*E* − 07	2.34*E* − 06	1.39*E* − 08	4.82*E* − 08	**0.00E + 00**	**0.00E + 00**
*F*2	7.16*E* + 05	4.42*E* + 05	2.62*E* + 06	2.16*E* + 06	5.11*E* + 04	4.09*E* + 04	3.07*E* + 05	2.59*E* + 05	7.28*E* + 05	1.16*E* + 06	**4.01E + 04**	**3.74E + 04**
*F*3	**0.00E + 00**	**0.00E + 00**	**0.00E + 00**	**0.00E + 00**	**0.00E + 00**	**0.00E + 00**	**0.00E + 00**	**0.00E + 00**	**0.00E + 00**	**0.00E + 00**	**0.00E + 00**	**0.00E + 00**
*F*4	7.16*E* + 03	2.30*E* + 03	5.31*E* + 03	1.98*E* + 03	**7.64E + 00**	**3.64E + 00**	1.04*E* + 03	6.49*E* + 02	1.55*E* + 03	2.11*E* + 03	5.52*E* + 02	4.35*E* + 02
*F*5	**0.00E + 00**	**0.00E + 00**	4.85*E* + 01	1.34*E* + 01	4.64*E* − 02	3.16*E* − 02	7.30*E* − 01	3.80*E* + 00	5.24*E* − 07	1.43*E* − 06	**0.00E + 00**	**0.00E + 00**
*F*6	5.71*E* + 00	4.78*E* + 00	2.03*E* + 01	2.04*E* + 01	7.76*E* + 00	3.97*E* + 00	2.09*E* + 01	2.60*E* + 01	2.82*E* + 01	3.25*E* + 01	**4.03E + 00**	**4.80E + 00**
*F*7	**0.00E + 00**	**0.00E+00**	**0.00E + 00**	**0.00E + 00**	**0.00E + 00**	**0.00E + 00**	**0.00E + 00**	**0.00E + 00**	**0.00E + 00**	**0.00E + 00**	**0.00E + 00**	**0.00E + 00**
*F*8	6.78*E* − 01	3.71*E* + 00	**4.44E − 16**	**3.01E − 31**	**4.44E − 16**	**3.01E − 31**	6.77*E* − 01	3.71*E* + 00	1.22*E* + 01	1.01*E* + 01	**4.44E − 16**	**3.01E − 31**
*F*9	**0.00E + 00**	**0.00E + 00**	**0.00E + 00**	**0.00E + 00**	**0.00E + 00**	**0.00E + 00**	**0.00E + 00**	**0.00E + 00**	**0.00E + 00**	**0.00E + 00**	**0.00E + 00**	**0.00E + 00**
*F*10	7.48*E* − 01	2.40*E* − 01	2.86*E* + 01	2.44*E* + 01	7.28*E* − 01	1.61*E* − 01	5.27*E* + 00	4.75E+00	5.90*E* +00	4.26*E* + 00	**1.31E − 01**	**8.01E − 02**
*F*11	**0.00E + 00**	**0.00E + 00**	**0.00E + 00**	**0.00E + 00**	**0.00E + 00**	**0.00E + 00**	**0.00E + 00**	**0.00E + 00**	**0.00E + 00**	**0.00E + 00**	**0.00E + 00**	**0.00E + 00**
*F*12	**0.00E + 00**	**0.00E + 00**	**0.00E + 00**	**0.00E + 00**	**0.00E + 00**	**0.00E + 00**	**0.00E + 00**	**0.00E + 00**	**0.00E + 00**	**0.00E + 00**	**0.00E + 00**	**0.00E + 00**
*F*13	**0.00E + 00**	**0.00E + 00**	**0.00E + 00**	**0.00E + 00**	**0.00E + 00**	**0.00E + 00**	**0.00E + 00**	**0.00E + 00**	**0.00E + 00**	**0.00E + 00**	**0.00E + 00**	**0.00E + 00**
*F*14	1.92*E* + 00	5.25*E* + 00	1.68*E* + 03	2.04*E* + 02	1.38*E* + 03	1.70*E* + 02	1.20*E* + 02	1.10*E* + 02	2.60*E* + 00	3.27*E* + 00	**7.04E − 01**	**1.56E + 00**
*F*15	6.26*E* + 02	1.55*E* + 02	1.54*E* + 03	1.68*E* + 02	1.03*E* + 03	1.78*E* + 02	5.33*E* + 02	2.85*E* + 02	7.31*E* + 02	2.81*E* + 02	**4.43E + 02**	**2.14E + 02**
*F*16	5.16*E* − 01	1.79*E* − 01	1.20*E* + 00	2.36*E* − 01	1.11*E* + 00	1.50*E* − 01	1.13*E* + 00	2.30*E* − 01	6.28*E* − 01	2.82*E* − 01	**4.10E − 01**	**1.85E − 01**
*F*17	4.98*E* + 00	5.10*E* + 00	7.16*E* + 01	1.88*E* + 01	3.12*E* + 01	5.59*E* + 00	6.15*E* + 00	4.54*E* + 00	4.89*E* + 00	5.12*E* + 00	**4.43E + 00**	**4.92E + 00**
*F*18	2.06*E* + 01	3.94*E* + 00	6.70*E* + 01	1.84*E* + 01	3.41*E* + 01	6.04*E* + 00	2.52*E* + 01	6.02*E* + 00	2.51*E* + 01	1.10*E* + 01	**1.79E + 01**	**5.21E + 00**
*F*19	**7.05E − 01**	**1.89E − 01**	5.42*E* + 00	1.34*E* + 00	2.23*E* + 00	3.18*E* − 01	8.89*E* − 01	2.04*E* − 01	1.65*E* + 00	1.01*E* + 00	8.08*E* − 01	2.49*E* − 01
*F*20	**0.00E + 00**	**0.00E + 00**	**0.00E + 00**	**0.00E + 00**	**0.00E + 00**	**0.00E + 00**	**0.00E + 00**	**0.00E + 00**	1.50*E* − 01	8.23*E* − 01	**0.00E + 00**	**0.00E + 00**
*F*21	**3.19E + 02**	**9.82E + 01**	4.09*E* + 02	2.50*E* + 01	4.00*E* + 02	2.56*E* − 04	3.84*E* + 02	5.14*E* + 01	3.98*E* + 02	7.01*E* + 00	3.90*E* + 02	5.59*E* + 01
*F*22	7.17*E* + 01	5.88*E* + 01	1.32*E* + 03	2.90*E* + 02	1.34*E* + 03	2.20*E* + 02	1.20*E* + 02	8.23*E* + 01	8.72*E* + 01	6.55*E* + 01	**6.54E + 01**	**6.12E + 01**
*F*23	6.37*E* + 02	1.59*E* + 02	1.65*E* + 03	2.05*E* + 02	1.43*E* + 03	1.52*E* + 02	**3.02E + 02**	**1.39E + 02**	8.88*E* + 02	3.61*E* + 02	3.96*E* + 02	2.06*E* + 02
*F*24	**1.00E + 02**	**8.14E − 03**	1.73*E* + 02	4.50*E* + 01	1.00*E* + 02	1.15*E* − 02	1.17*E* + 02	3.79*E* + 01	1.69*E* + 02	4.73*E* + 01	1.50*E* + 02	5.09*E* + 01
*F*25	1.00*E* + 02	1.28*E* − 04	1.17*E* + 02	3.76*E* + 01	1.01*E* + 02	1.41*E* − 01	1.03*E* + 02	1.98*E* + 00	1.00*E* + 02	1.08*E* − 04	**1.00E + 02**	**0.00E + 00**
*F*26	1.00*E* + 02	4.96*E* − 13	1.17*E* + 02	3.79*E* + 01	**1.00E + 02**	**4.28E − 13**	1.00*E* + 02	4.65*E* − 12	1.23*E* + 02	4.30*E* + 01	1.20*E* + 02	4.07*E* + 01
*F*27	3.09*E* + 02	3.35*E* − 01	3.16*E* + 02	4.02*E* + 01	**3.08E + 02**	**1.45E − 01**	3.10*E* + 02	5.89*E* − 01	3.21*E* + 02	4.33*E* + 01	3.09*E* + 02	3.19*E* − 01
*F*28	**3.31E + 02**	**2.48E + 02**	6.65*E* + 02	1.29*E* + 02	3.37*E* + 02	2.77*E* + 02	4.43*E* + 02	3.01*E* + 02	5.18*E* + 02	2.82*E* + 02	5.06*E* + 02	2.53*E* + 02

Bold indicates the best results obtained on each function.

**Table 9:** Data result of INCCLA with other algorithms on the 30-dimensional CEC2013 test suite.

Fun.	NSABC		MSCA		IATTP		ICSA		NCCLA		INCCLA	
	Mean	Std	Mean	Std	Mean	Std	Mean	Std	Mean	Std	Mean	Std
*F*1	**0.00E** **+** **00**	**0.00E** **+** **00**	9.60*E* **+** 03	4.32*E* **+** 03	6.24*E* **+** 00	3.00*E* **+** 00	3.36*E* **+** 01	3.41*E* **+** 01	1.99*E* − 05	5.60*E* − 05	**0.00E** **+** **00**	**0.00E** **+** **00**
*F*2	1.01*E* **+** 07	3.38*E* **+** 06	7.18*E* **+** 07	2.22*E* **+** 07	1.15*E* **+** 07	3.71*E* **+** 06	2.11*E* **+** 07	1.04*E* **+** 07	7.59*E* **+** 06	4.32*E* **+** 06	**8.10E** **+** **05**	**4.96E** **+** **05**
*F*3	**0.00E** **+** **00**	**0.00E** **+** **00**	**0.00E** **+** **00**	**0.00E** **+** **00**	**0.00E** **+** **00**	**0.00E** **+** **00**	**0.00E** **+** **00**	**0.00E** **+** **00**	**0.00E** **+** **00**	**0.00E** **+** **00**	**0.00E** **+** **00**	**0.00E** **+** **00**
*F*4	8.13*E* **+** 04	1.31*E* **+** 04	3.74*E* **+** 04	7.65*E* **+** 03	**9.60E** **+** **02**	**4.01E** **+** **02**	1.33*E* **+** 04	2.91*E* **+** 03	7.59*E* **+** 03	2.43*E* **+** 03	1.10*E* **+** 04	3.46*E* **+** 03
*F*5	**0.00E** **+** **00**	**0.00E** **+** **00**	2.72*E* **+** 03	1.54*E* **+** 03	1.58*E* **+** 01	9.80*E* **+** 00	3.09*E* **+** 02	2.74*E* **+** 02	8.91*E* − 04	3.77*E* − 03	**0.00E** **+** **00**	**0.00E** **+** **00**
*F*6	**2.27E** **+** **01**	**1.20E** **+** **01**	6.45*E* **+** 02	3.67*E* **+** 02	8.24*E* **+** 01	2.61*E* **+** 01	1.35*E* **+** 02	3.38*E* **+** 01	6.64*E* **+** 01	3.21*E* **+** 01	2.40*E* **+** 01	2.04*E* **+** 01
*F*7	**0.00E** **+** **00**	**0.00E** **+** **00**	8.51*E* − 02	3.51*E* − 01	**0.00E** **+** **00**	**0.00E** **+** **00**	**0.00E** **+** **00**	**0.00E** **+** **00**	**0.00E** **+** **00**	**0.00E** **+** **00**	**0.00E** **+** **00**	**0.00E** **+** **00**
*F*8	2.10*E* **+** 01	5.54*E* − 02	2.10*E* **+** 01	5.62*E* − 02	2.10*E* **+** 01	5.72*E* − 02	2.10*E* **+** 01	6.35*E* − 02	2.10E − 01	5.25*E* − 02	**2.10E** **+** **01**	**5.23E** − **02**
*F*9	**0.00E** **+** **00**	**0.00E** **+** **00**	2.37*E* **+** 00	6.82*E* **+** 00	**0.00E** **+** **00**	**0.00E** **+** **00**	**0.00E** **+** **00**	**0.00E** **+** **00**	5.26*E* **+** 00	9.82*E* **+** 00	**0.00E** **+** **00**	**0.00E** **+** **00**
*F*10	2.20*E* **+** 00	4.88*E* − 01	1.06*E* **+** 03	2.58*E* **+** 02	2.14*E* **+** 01	1.00*E* **+** 01	1.56*E*+02	7.69*E*+01	9.26*E*+00	7.28*E*+00	**2.10*E*−01**	**5.91*E*−02**
*F*11	**0.00E** **+** **00**	**0.00E** **+** **00**	**0.00E** **+** **00**	**0.00E** **+** **00**	**0.00E** **+** **00**	**0.00E** **+** **00**	1.99*E* − 01	7.57*E* − 01	**0.00E** **+** **00**	**0.00E** **+** **00**	**0.00E** **+** **00**	**0.00E** **+** **00**
*F*12	2.03*E* **+** 01	4.62*E* **+** 01	3.05*E* **+** 01	6.95*E* **+** 01	**0.00E** **+** **00**	**0.00E** **+** **00**	**0.00E** **+** **00**	**0.00E** **+** **00**	1.16*E* **+** 02	3.57*E* **+** 01	**0.00E** **+** **00**	**0.00E** **+** **00**
*F*13	8.17*E* **+** 00	3.11*E* **+** 01	4.51*E* **+** 01	8.33*E* **+** 01	**0.00E** **+** **00**	**0.00E** **+** **00**	**0.00E** **+** **00**	**0.00E** **+** **00**	1.31*E* **+** 02	6.87*E* **+** 01	**0.00E** **+** **00**	**0.00E** **+** **00**
*F*14	6.38*E* **+** 00	2.25*E* **+** 01	7.02*E* **+** 03	4.08*E* **+** 02	6.87*E* **+** 03	4.40*E* **+** 02	2.73*E* **+** 03	6.75*E* **+** 02	1.78*E* **+** 01	3.12*E* **+** 01	**6.29E** **+** **00**	**4.92E** **+** **00**
*F*15	3.99*E* **+** 03	3.54*E* **+** 02	7.97*E* **+** 03	2.26*E* **+** 02	6.90*E* **+** 03	5.19*E* **+** 02	6.11*E* **+** 03	1.01*E* **+** 03	4.79*E* **+** 03	1.50*E* **+** 03	**3.94E** **+** **03**	**6.65E** **+** **02**
*F*16	1.08*E* **+** 00	2.70*E* − 01	2.79*E* **+** 00	2.88*E* − 01	2.57*E* **+** 00	3.39*E* − 01	2.60*E* **+** 00	2.71*E* − 01	2.68*E* **+** 00	3.22*E* − 01	**9.33E** − **01**	**2.63E** − **01**
*F*17	6.77*E* **+** 00	1.19*E* **+** 01	6.47*E* **+** 02	1.18*E* **+** 02	2.05*E* **+** 02	1.91*E* **+** 01	9.80*E* **+** 01	3.07*E* **+** 01	9.59*E* **+** 00	1.21*E* **+** 01	**5.43E** **+** **00**	**7.92E** **+** **00**
*F*18	1.66*E* **+** 02	2.57*E* **+** 01	6.17*E* **+** 02	1.94*E* **+** 02	2.21*E* **+** 02	1.78*E* **+** 01	2.22*E* **+** 02	3.41*E* **+** 01	1.77*E* **+** 02	4.90*E* **+** 01	**9.65E** **+** **01**	**2.06E** **+** **01**
*F*19	8.23*E* **+** 00	1.70*E* **+** 00	3.10*E* **+** 03	4.81*E* **+** 03	1.73*E* **+** 01	9.95*E* − 01	1.58*E* **+** 01	8.31*E* **+** 00	1.57*E* **+** 01	7.70*E* **+** 00	**5.32E** **+** **00**	**2.09E** **+** **00**
*F*20	8.44*E* **+** 00	6.04*E* **+** 00	3.10*E* **+** 00	5.26*E* **+** 00	5.56*E* − 01	2.13*E* **+** 00	6.58*E* **+** 00	4.69*E* **+** 00	1.31*E* **+** 01	3.16*E* **+** 00	**0.00E** **+** **00**	**0.00E** **+** **00**
*F*21	**3.97E** **+** **02**	**1.69E** **+** **01**	1.01*E* **+** 03	2.52*E* **+** 02	4.02*E* **+** 02	5.22*E* − 01	4.16*E* **+** 02	2.11*E* **+** 01	4.00*E* **+** 02	2.73*E* − 01	4.00*E* **+** 02	0.00*E* **+** 00
*F*22	8.12*E* **+** 01	6.21*E* **+** 01	7.45*E* **+** 03	5.44*E* **+** 02	7.20*E* **+** 03	3.25*E* **+** 02	1.99*E* **+** 03	7.62*E* **+** 02	1.17*E* **+** 02	6.11*E* **+** 01	**7.70E** **+** **01**	**5.90E** **+** **01**
*F*23	4.40*E* **+** 03	3.98*E* **+** 02	7.87*E* **+** 03	3.16*E* **+** 02	7.60*E* **+** 03	4.00*E* **+** 02	5.40*E* **+** 03	1.21*E* **+** 03	4.21*E* **+** 03	6.46*E* **+** 02	**4.06E** **+** **03**	**5.45E** **+** **02**
*F*24	2.00*E* **+** 02	4.34*E* − 02	2.07*E* **+** 02	1.04*E* **+** 01	2.00*E* **+** 02	9.22*E* − 02	2.01*E* **+** 02	2.95*E* − 01	2.04*E* **+** 02	1.37*E* **+** 01	**2.00E** **+** **02**	**2.44E** − **02**
*F*25	**2.27E** **+** **02**	**2.13E** **+** **01**	2.78*E* **+** 02	3.44*E* **+** 01	2.42*E* **+** 02	3.48*E* **+** 01	2.82*E* **+** 02	2.12*E* **+** 01	2.88*E* **+** 02	3.40*E* **+** 01	2.40*E* **+** 02	3.15*E* **+** 01
*F*26	**2.01E** **+** **02**	**1.77E** − **01**	3.06*E* **+** 02	5.46*E* **+** 01	2.58*E* **+** 02	4.81*E* **+** 01	2.91*E* **+** 02	3.01*E* **+** 01	3.08*E* **+** 02	4.25*E* **+** 01	2.87*E* **+** 02	3.45*E* **+** 01
*F*27	3.31*E* **+** 02	2.04*E* **+** 01	6.23*E* **+** 02	2.42*E* **+** 02	3.37*E* **+** 02	9.82*E* **+** 01	3.57*E* **+** 02	8.59*E* **+** 01	4.46*E* **+** 02	2.75*E* **+** 02	**3.13E** **+** **02**	**8.90E** − **01**
*F*28	9.39*E* **+** 02	1.59*E* **+** 02	2.58*E* **+** 03	4.31*E* **+** 02	1.01*E* **+** 03	2.17*E* **+** 01	1.60*E* **+** 03	3.69*E* **+** 02	1.46*E* **+** 03	8.95*E* **+** 02	**9.14E** **+** **02**	**2.15E** **+** **01**

Bold indicates the best results obtained on each function.

**Table 10:** Data result of INCCLA with other algorithms on the 100-dimensional CEC2013 test suite.

Fun.	NSABC		MSCA		IATTP		ICSA		NCCLA		INCCLA	
	Mean	Std	Mean	Std	Mean	Std	Mean	Std	Mean	Std	Mean	Std
*F*1	**1.85E** − **20**	**2.55E** − **20**	8.85*E* **+** 04	9.37*E* **+** 03	1.73*E* **+** 03	2.84*E* **+** 02	1.36*E* **+** 04	3.64*E* **+** 03	1.15*E*+00	1.85*E* **+** 00	7.80*E* − 12	1.18*E* − 11
*F*2	6.23*E* **+** 07	1.21*E* **+** 07	9.81*E* **+** 08	2.70*E* **+** 08	2.20*E* **+** 08	4.82*E* **+** 07	2.20*E* **+** 08	7.15*E* **+** 07	3.58*E* **+** 07	8.52*E* **+** 06	**2.02E** **+** **07**	**4.71E** **+** **06**
*F*3	**0.00E** **+** **00**	**0.00E** **+** **00**	1.28*E* **+** 15	3.11*E* **+** 15	1.53*E* **+** 10	2.34*E* **+** 10	7.89*E* **+** 11	1.45*E* **+** 12	**0.00E** **+** **00**	**0.00E** **+** **00**	**0.00E** **+** **00**	**0.00E** **+** **00**
*F*4	3.11*E* **+** 05	3.36*E* **+** 04	2.21*E* **+** 05	1.57*E* **+** 04	**3.95E** **+** **04**	**6.28E** **+** **03**	9.43*E* **+** 04	1.66*E* **+** 04	6.76*E* **+** 04	1.36*E* **+** 04	1.19*E* **+** 05	1.52*E* **+** 04
*F*5	**2.19E** − **12**	**2.45E** − **12**	4.07*E* **+** 04	1.22*E* **+** 04	1.63*E* **+** 03	2.17*E* **+** 02	8.53*E* **+** 03	3.07*E* **+** 03	1.81*E* **+** 00	4.28*E* **+** 00	1.74*E* − 06	1.22*E* − 06
*F*6	**2.27E** **+** **02**	**3.41E** **+** **01**	1.37*E* **+** 04	2.93*E* **+** 03	8.88*E* **+** 02	1.28*E* **+** 02	2.03*E* **+** 03	3.77*E* **+** 02	3.20*E* **+** 02	5.22*E* **+** 01	2.36*E* **+** 02	5.69*E* **+** 01
*F*7	4.26*E* **+** 02	2.99*E* **+** 02	1.26*E* **+** 04	9.57*E* **+** 03	2.49*E* **+** 02	1.51*E* **+** 02	5.76*E*+02	4.53*E*+02	3.93*E*+02	4.94*E*+02	**0.00*E*+00**	**0.00E+00**
*F*8	2.13*E*+01	2.11*E* − 02	2.13*E*+01	3.44*E* − 02	**2.13*E*+01**	**1.82E** − **02**	2.13*E*+01	2.34*E*−02	2.13*E*+01	2.89*E*−02	2.13*E*+01	2.14*E*−02
*F*9	1.28*E* **+** 02	3.51*E* **+** 00	1.24*E* **+** 02	8.02*E* **+** 00	1.18*E* **+** 02	6.41*E* **+** 00	7.86*E* **+** 01	1.05*E* **+** 01	1.01*E* **+** 02	8.79*E* **+** 00	**7.02E** **+** **01**	**3.63E** **+** **01**
*F*10	2.49*E* **+** 01	1.08*E* **+** 01	9.81*E* **+** 03	1.29*E* **+** 03	1.41*E* **+** 03	2.26*E* **+** 02	2.29*E* **+** 03	4.02*E* **+** 02	1.60*E* **+** 02	4.54*E* **+** 01	**4.63E** **+** **00**	**1.45E** **+** **00**
*F*11	**0.00E** **+** **00**	**0.00E** **+** **00**	**0.00E** **+** **00**	**0.00E** **+** **00**	6.96*E* − 01	3.81*E* **+** 00	8.47*E* **+** 01	2.79*E* **+** 01	**0.00E** **+** **00**	**0.00E** **+** **00**	**0.00E** **+** **00**	**0.00E** **+** **00**
*F*12	8.02*E* **+** 02	7.60*E* **+** 01	1.25*E* **+** 03	1.38*E* **+** 02	7.08*E* **+** 02	7.86*E* **+** 01	5.77*E* **+** 02	7.69*E* **+** 01	5.71*E* **+** 02	1.02*E* **+** 02	**5.21E** **+** **02**	**7.37 ** *E* **+** **01**
*F*13	9.18*E* **+** 02	7.95*E* **+** 01	1.22*E* **+** 03	1.55*E* **+** 02	6.97*E* **+** 02	6.93*E* **+** 01	6.27*E* **+** 02	4.48*E* **+** 01	8.15*E* **+** 02	1.51*E* **+** 02	**6.24E** **+** **02**	**4.86E** **+** **01**
*F*14	**1.80E** **+** **02**	**1.49E** **+** **02**	3.14*E* **+** 04	7.61*E* **+** 02	3.15*E* **+** 04	1.24*E* **+** 03	1.89*E* **+** 04	2.67*E* **+** 03	2.65*E* **+** 02	2.15*E* **+** 02	7.58*E* **+** 03	5.27*E* **+** 03
*F*15	**1.80E** **+** **04**	**9.42E** **+** **02**	3.21*E* **+** 04	5.71*E* **+** 02	3.10*E* **+** 04	6.01*E* **+** 02	3.05*E* **+** 04	5.18*E* **+** 02	3.01*E* **+** 04	2.86*E* **+** 03	2.03*E* **+** 04	1.71*E* **+** 03
*F*16	2.56*E* **+** 00	3.13*E* − 01	4.53*E* **+** 00	2.88*E* − 01	4.36*E* **+** 00	2.58*E* − 01	4.30*E* **+** 00	2.67*E* − 01	4.27*E* **+** 00	2.93*E* − 01	**2.06E + 00**	**3.75*E*−01**
*F*17	**4.28E** **+** **00**	**9.78E** **+** **00**	4.72*E* **+** 03	3.43*E* **+** 02	1.31*E* **+** 03	7.39*E* **+** 01	1.28*E* **+** 03	2.28*E* **+** 02	4.60*E* **+** 01	8.90*E* **+** 00	9.60*E* **+** 01	2.45*E* **+** 01
*F*18	1.75*E* **+** 03	1.44*E* **+** 02	4.90*E* **+** 03	4.89*E* **+** 02	1.32*E* **+** 03	8.63*E* **+** 01	1.74*E* **+** 03	1.58*E* **+** 02	1.14*E* **+** 03	2.04*E* **+** 02	**7.03E** **+** **02**	**1.24E** **+** **02**
*F*19	1.10*E* **+** 02	1.27*E* **+** 01	4.60*E* **+** 05	1.90*E* **+** 05	6.99*E* **+** 02	2.81*E* **+** 02	7.19*E* **+** 03	4.08*E* **+** 03	1.80*E* **+** 02	4.93*E* **+** 01	**7.04E** **+** **01**	**1.88E** **+** **01**
*F*20	5.00*E* **+** 01	0.00*E* **+** 00	5.00*E* **+** 01	0.00*E* **+** 00	5.00*E* **+** 01	2.63*E* − 09	5.00*E* **+** 01	1.50*E* − 04	5.00*E* **+** 01	1.83*E* − 02	**4.99E** **+** **01**	**1.65E** − **01**
*F*21	3.79*E* **+** 02	3.43*E* **+** 01	7.31*E* **+** 03	2.84*E* **+** 02	1.29*E* **+** 03	4.26*E* **+** 02	5.05*E* **+** 03	7.92*E* **+** 02	4.46*E* **+** 02	6.81*E* **+** 00	**3.49E** **+** **02**	**4.88E** **+** **01**
*F*22	**2.54E** **+** **02**	**1.24E** **+** **02**	3.16*E* **+** 04	6.60*E* **+** 02	3.11*E* **+** 04	1.33*E* **+** 03	1.78*E* **+** 04	3.63*E* **+** 03	2.89*E* **+** 02	1.27*E* **+** 02	7.59*E* **+** 03	6.74*E* **+** 03
*F*23	2.23*E* **+** 04	1.73*E* **+** 03	3.35*E* **+** 04	6.13*E* **+** 02	3.31*E* **+** 04	6.55*E* **+** 02	3.07*E* **+** 04	8.30*E* **+** 02	3.11*E* **+** 04	3.75*E* **+** 03	**2.22E** **+** **04**	**1.48E** **+** **03**
*F*24	4.72*E* **+** 02	7.75*E* **+** 01	5.65*E* **+** 02	4.14*E* **+** 01	4.40*E* **+** 02	6.67*E* **+** 01	4.12*E* **+** 02	3.62*E* **+** 01	4.06*E* **+** 02	1.25*E* **+** 02	**2.42E** **+** **02**	**8.01E** **+** **01**
*F*25	6.06*E* **+** 02	1.35*E* **+** 01	6.73*E* **+** 02	2.88*E* **+** 01	5.57*E* **+** 02	1.70*E* **+** 01	5.51*E* **+** 02	1.74*E* **+** 01	5.76*E* **+** 02	2.28*E* **+** 01	**5.09E** **+** **02**	**4.82E** **+** **01**
*F*26	**2.19E** **+** **02**	**7.44E** **+** **01**	5.45*E* **+** 02	4.62*E* **+** 01	4.52*E* **+** 02	1.06*E* **+** 02	4.27*E* **+** 02	5.66*E* **+** 01	4.47*E* **+** 02	9.21*E* **+** 01	3.10*E* **+** 02	3.85*E* **+** 01
*F*27	3.30*E* **+** 03	2.41*E* **+** 02	3.30*E* **+** 03	4.34*E* **+** 02	2.49*E* **+** 03	6.09*E* **+** 02	1.97*E* **+** 03	4.12*E* **+** 02	2.16*E* **+** 03	7.89*E* **+** 02	**5.76E** **+** **02**	**5.95E** **+** **02**
*F*28	4.58*E* **+** 03	1.28*E* **+** 03	1.47*E* **+** 04	1.01*E* **+** 03	9.16*E* **+** 03	3.02*E* **+** 03	1.02*E* **+** 04	1.02*E* **+** 03	7.16*E* **+** 03	3.07*E* **+** 03	**4.08E** **+** **03**	**1.19E** **+** **03**

Bold indicates the best results obtained on each function.

**Table 11:** Wilcoxon rank sum test results of INCCLA with other algorithms on the 10-dimensional and 30-dimensional CEC2013 test suite.

Function	*D* = 10 *p* value (vs.INCCLA)					*D* = 30 *p* value (vs.INCCLA)					*D* = 100 *p* value (vs.INCCLA)				
	NSABC	MSCA	IATTP	ICSA	NCCLA	NSABC	MSCA	IATTP	ICSA	NCCLA	NSABC	MSCA	IATTP	ICSA	NCCLA
*F*1	1.000 (=)	0.000 (−)	0.000 (−)	0.000 (−)	0.000 (−)	1.000 (=)	0.000 (−)	0.000 (−)	0.000 (−)	0.000 (−)	0.000 (+)	0.000 (−)	0.000 (−)	0.000 (−)	0.000 (−)
*F*2	0.000 (−)	0.000 (−)	0.290 (=)	0.000 (−)	0.000 (−)	0.000 (−)	0.000 (−)	0.000 (−)	0.000 (−)	0.000 (−)	0.000 (−)	0.000 (−)	0.000 (−)	0.000 (−)	0.000 (−)
*F*3	1.000 (=)	1.000 (=)	1.000 (=)	1.000 (=)	1.000 (=)	1.000 (=)	1.000 (=)	1.000 (=)	1.000 (=)	1.000 (=)	1.000 (=)	0.000 (−)	0.000 (−)	0.000 (−)	1.000 (=)
*F*4	0.000 (−)	0.000 (−)	0.000 (+)	0.000 (−)	0.002 (−)	0.000 (−)	0.000 (−)	0.000 (+)	0.004 (−)	0.000 (+)	0.000 (−)	0.000 (−)	0.000 (+)	0.000 (+)	0.000 (+)
*F*5	1.000 (=)	0.000 (−)	0.000 (−)	0.000 (−)	0.000 (−)	1.000 (=)	0.000 (−)	0.000 (−)	0.000 (−)	0.000 (−)	0.000 (+)	0.000 (−)	0.000 (−)	0.000 (−)	0.000 (−)
*F*6	0.030 (−)	0.000 (−)	0.000 (−)	0.000 (−)	0.000 (−)	0.000 (+)	0.000 (−)	0.000 (−)	0.000 (−)	0.000 (−)	0.190 (=)	0.000 (−)	0.000 (−)	0.000 (−)	0.000 (−)
*F*7	1.000 (=)	1.000 (=)	1.000 (=)	1.000 (=)	1.000 (=)	1.000 (=)	0.160 (=)	1.000 (=)	1.000 (=)	1.000 (=)	0.000 (−)	0.000 (−)	0.000 (−)	0.000 (−)	0.000 (−)
*F*8	0.333 (=)	1.000 (=)	1.000 (=)	0.333 (=)	0.000 (−)	0.865 (=)	0.935 (=)	0.258 (=)	0.654 (=)	0.695 (=)	0.970 (=)	0.137 (=)	0.728 (=)	0.180 (=)	0.911 (=)
*F*9	1.000 (=)	1.000 (=)	1.000 (=)	1.000 (=)	1.000 (=)	1.000 (=)	0.011 (−)	1.000 (=)	1.000 (=)	0.005 (−)	0.000 (−)	0.000 (−)	0.000 (−)	0.200 (=)	0.000 (−)
*F*10	0.000 (−)	0.000 (−)	0.000 (−)	0.000 (−)	0.000 (−)	0.000 (−)	0.000 (−)	0.000 (−)	0.000 (−)	0.000 (−)	0.000 (−)	0.000 (−)	0.000 (−)	0.000 (−)	0.000 (−)
*F*11	1.000 (=)	1.000 (=)	1.000 (=)	1.000 (=)	1.000 (=)	1.000 (=)	1.000 (=)	1.000 (=)	0.081 (=)	1.000 (=)	1.000 (=)	1.000 (=)	0.333 (=)	0.000 (−)	1.000 (=)
*F*12	1.000 (=)	1.000 (=)	1.000 (=)	1.000 (=)	1.000 (=)	0.021 (−)	0.021 (−)	1.000 (=)	1.000 (=)	0.000 (−)	0.000 (−)	0.000 (−)	0.000 (−)	0.006 (−)	0.065 (=)
*F*13	1.000 (=)	1.000 (=)	1.000 (=)	1.000 (=)	1.000 (=)	0.160 (=)	0.002 (−)	1.000 (=)	1.000 (=)	0.000 (−)	0.000 (−)	0.000 (−)	0.000 (−)	0.706 (=)	0.000 (−)
*F*14	0.745 (=)	0.000 (−)	0.000 (−)	0.000 (−)	0.000 (−)	0.000 (−)	0.000 (−)	0.000 (−)	0.000 (−)	0.004 (−)	0.000 (+)	0.000 (−)	0.000 (−)	0.000 (−)	0.000 (+)
*F*15	0.000 (−)	0.000 (−)	0.000 (−)	0.195 (=)	0.000 (−)	0.807 (=)	0.000 (−)	0.000 (−)	0.000 (−)	0.039 (−)	0.000 (+)	0.000 (−)	0.000 (−)	0.000 (−)	0.000 (−)
*F*16	0.030 (−)	0.000 (−)	0.000 (−)	0.000 (−)	0.002 (−)	0.046 (−)	0.000 (−)	0.000 (−)	0.000 (−)	0.000 (−)	0.000 (−)	0.000 (−)	0.000 (−)	0.000 (−)	0.000 (−)
*F*17	0.075 (=)	0.000 (−)	0.000 (−)	0.037 (−)	0.176 (=)	0.000 (−)	0.000 (−)	0.000 (−)	0.000 (−)	0.007 (−)	0.000 (+)	0.000 (−)	0.000 (−)	0.000 (−)	0.000 (+)
*F*18	0.015 (−)	0.000 (−)	0.000 (−)	0.000 (−)	0.004 (−)	0.000 (−)	0.000 (−)	0.000 (−)	0.000 (−)	0.000 (−)	0.000 (−)	0.000 (−)	0.000 (−)	0.000 (−)	0.000 (−)
*F*19	0.055 (=)	0.000 (−)	0.000 (−)	0.411 (=)	0.000 (−)	0.000 (−)	0.000 (−)	0.000 (−)	0.000 (−)	0.000 (−)	0.000 (−)	0.000 (−)	0.000 (−)	0.000 (−)	0.000 (−)
*F*20	1.000 (=)	1.000 (=)	1.000 (=)	1.000 (=)	0.333 (=)	0.000 (−)	0.002 (−)	0.160 (=)	0.000 (−)	0.000 (−)	0.041 (−)	0.041 (−)	0.151 (=)	0.151 (=)	0.043 (−)
*F*21	0.001 (+)	0.000 (−)	0.000 (−)	0.038 (−)	0.000 (−)	0.333 (=)	0.000 (−)	0.000 (−)	0.000 (−)	0.000 (−)	0.000 (−)	0.000 (−)	0.000 (−)	0.000 (−)	0.000 (−)
*F*22	0.711 (=)	0.000 (−)	0.000 (−)	0.001 (−)	0.013 (−)	0.166 (=)	0.000 (−)	0.000 (−)	0.000 (−)	0.028 (−)	0.000 (+)	0.000 (−)	0.000 (−)	0.000 (−)	0.000 (+)
*F*23	0.000 (−)	0.000 (−)	0.000 (−)	0.102 (=)	0.000 (−)	0.011 (−)	0.000 (−)	0.000 (−)	0.000 (−)	0.297 (=)	0.652 (=)	0.000 (−)	0.000 (−)	0.000 (−)	0.000 (−)
*F*24	0.003 (+)	0.000 (−)	0.061 (=)	0.395 (=)	0.000 (−)	0.000 (−)	0.000 (−)	0.000 (−)	0.000 (−)	0.000 (−)	0.000 (−)	0.000 (−)	0.000 (−)	0.000 (−)	0.000 (−)
*F*25	0.000 (−)	0.000 (−)	0.000 (−)	0.000 (−)	0.000 (−)	0.888 (=)	0.000 (−)	0.455 (=)	0.000 (−)	0.000 (−)	0.000 (−)	0.000 (−)	0.000 (−)	0.000 (−)	0.000 (−)
*F*26	0.011 (+)	1.000 (=)	0.011 (+)	0.011 (+)	0.479 (=)	0.000 (+)	0.000 (−)	0.911 (=)	0.000 (−)	0.000 (−)	0.000 (+)	0.000 (−)	0.000 (−)	0.000 (−)	0.000 (−)
*F*27	0.000 (−)	0.000 (−)	0.000 (+)	0.000 (−)	0.000 (−)	0.000 (−)	0.000 (−)	0.000 (−)	0.000 (−)	0.000 (−)	0.000 (−)	0.000 (−)	0.000 (−)	0.000 (−)	0.000 (−)
*F*28	0.002 (+)	0.000 (−)	0.317 (=)	0.771 (=)	0.055 (=)	0.000 (−)	0.000 (−)	0.000 (−)	0.000 (−)	0.000 (−)	0.000 (−)	0.000 (−)	0.000 (−)	0.000 (−)	0.000 (−)
+/ = /−	4/14/10	0/9/19	3/11/14	1/13/14	0/10/18	2/12/14	0/4/24	1/10/17	0/7/21	1/5/22	7/5/16	0/2/26	1/3/24	1/4/23	4/4/20

**Table 12:** Friedman test results of 6 algorithms.

Dimension		NSABC	MSCA	IATTP	ICSA	NCCLA	INCCLA
*D* = 10	Avg.rank	2.68	4.96	3.54	3.50	4.07	2.25
	sort	2	6	3	4	5	1

*D* = 30	Avg.rank	2.50	5.34	3.57	4.07	3.73	1.79
	sort	2	6	3	5	4	1

*D* = 100	Avg.rank	2.91	5.59	4.04	3.93	2.86	1.68
	sort	3	6	5	4	2	1

**Table 13:** Data result of INCCLA with other algorithms on the CEC2020 test suite.

Function	NSABC		MSCA		IATTP		ICSA		NCCLA		INCCLA
	Mean (std)	*p* value (vs. INCCLA)	Mean (std)	*p* value (vs. INCCLA)	Mean (std)	*p* value (vs. INCCLA)	Mean (std)	*p* value (vs. INCCLA)	Mean (std)	*p* value (vs. INCCLA)	Mean (std)
*F*1	1.53*E* + 03(1.89*E* + 03)	0.000 (−)	1.42*E* + 08 (9.70*E* + 07)	0.000 (−)	2.66*E* + 04 (1.66*E* + 04)	0.000 (−)	4.17*E* + 04 (1.28*E* + 05)	0.000 (−)	3.25*E* + 03 (2.75*E* + 03)	0.000 (−)	**2.38E** − **01 (5.98E** − **01)**
*F*2	**7.31E** + **01 (6.93E** + **01)**	0.739 (=)	1.15*E* + 03 (2.35*E* + 02)	0.000 (−)	1.17*E* + 03 (1.42*E* + 02)	0.000 (−)	1.71*E* + 02 (1.47*E* + 02)	0.145 (=)	3.23*E* + 02 (2.38*E* + 02)	0.000 (−)	9.33*E* + 01(8.63*E* + 01)
*F*3	**1.25E** + **01 (1.87E** + **00)**	0.000 (+)	5.63*E* + 01 (9.38*E* + 00)	0.000 (−)	4.01*E* + 01 (4.60*E* + 00)	0.000 (−)	1.53*E* + 01 (2.38*E* + 00)	0.112 (=)	3.12*E* + 01 (7.79*E* + 00)	0.000 (−)	1.63*E* + 01(3.44*E* + 00)
*F*4	6.49*E* − 01 (1.19*E* − 01)	0.684 (=)	7.65*E* + 00 (2.43*E* + 00)	0.000 (−)	2.03*E* + 00 (3.89*E* − 01)	0.000 (−)	5.21*E* + 00 (1.86*E* + 01)	0.008 (−)	1.28*E* + 00 (5.88*E* − 01)	0.000 (−)	**6.20E** − **01 (2.53E** − **01)**
*F*5	3.53*E* + 04 (2.75*E* + 04)	0.000 (−)	9.21*E* + 03 (6.13*E* + 03)	0.000 (−)	4.94*E* + 02 (2.68*E* + 02)	0.000 (−)	4.68*E* + 03 (1.74*E* + 04)	0.000 (−)	6.71*E* + 03 (1.07*E* + 04)	0.000 (−)	**1.34E** + **02 (1.04E** + **02)**
*F*6	**2.03E** + **01 (4.13E** + **01)**	0.994 (=)	1.21*E* + 02 (5.85*E* + 01)	0.000 (−)	4.16*E* + 01 (4.74*E* + 01)	0.011 (+)	4.63*E* + 01 (6.54*E* + 01)	0.008 (−)	1.17*E* + 02 (8.56*E* + 01)	0.000 (−)	4.53*E* + 01(6.66*E* + 01)
*F*7	4.11*E* + 03 (3.95*E* + 03)	0.000 (−)	2.83*E* + 03 (1.39*E* + 03)	0.000 (−)	1.42*E* + 02 (6.70*E* + 01)	0.000 (−)	1.02*E* + 02 (8.29*E* + 01)	0.000 (−)	4.84*E* + 03 (5.59*E* + 03)	0.000 (−)	**2.86E** + **01 (3.67E** + **01)**
*F*8	1.07*E* + 02 (1.49*E* + 01)	0.570 (=)	1.21*E* + 02 (6.45*E* + 00)	0.000 (−)	1.07*E* + 02 (1.52*E* + 01)	0.000 (−)	1.10*E* + 02 (2.20*E* − 01)	0.000 (−)	1.10*E* + 02 (1.10*E* − 04)	0.000 (−)	**1.04E** + **02 (2.43E** + **01)**
*F*9	2.41*E* + 02 (1.10*E* + 02)	0.000 (+)	3.74*E* + 02 (6.78*E* + 00)	0.000 (−)	**2.08E** + **02 (1.18E** + **02)**	0.007 (+)	3.13*E* + 02 (7.19*E* + 01)	0.013 (+)	3.47*E* + 02 (6.53*E* + 00)	0.001 (−)	3.18*E* + 02 (7.44*E* + 01)
*F*10	4.15*E* + 02 (2.27*E* + 01)	0.100 (=)	4.33*E* + 02 (2.81*E* + 01)	0.000 (−)	4.17*E* + 02 (2.25*E* + 01)	0.610 (=)	4.31*E* + 02 (2.23*E* + 01)	0.000 (−)	4.18*E* + 02 (2.33*E* + 01)	0.085 (=)	**4.14E** + **02 (2.21E** + **01)**
+/=/−	2/5/3		0/0/10		2/1/7		1/2/7		0/1/9		
Avg.rank	2.45		5.60		3.25		3.65		4.25		1.80
Sort	2		6		3		4		5		1

## Data Availability

The labeled datasets used to support the findings of this study are available from the corresponding author upon request.
